The article "Connectedness in cross-assets and digital assets attention indices" was published in 2023. Journal: Heliyon.

# Connectedness in cross-assets and digital assets attention indices

**DOI:** 10.1016/j.heliyon.2023.e20668

**Published:** 2023-10-11

**Authors:** Zynobia Barson, Peterson Owusu Junior

**Affiliations:** Department of Finance, School of Business, University of Cape Coast, Cape Coast, Ghana

**Keywords:** NFTAI, ICEA, CBDCAI, Spillover, Frequency-domain

## Abstract

We explore both the static and dynamic connectedness across traditional and unconventional assets classes using the Baruník-Křehlík connectedness and wavelets techniques. These techniques are used to characterise the static and rolling-window connectedness of 12 conventional assets and Non-Fungible Tokens (NFT), Index On Cryptocurrency Environmental Attention (ICEA) and Central Bank Digital Currency (CBDC) attention indices. Between January 25, 2010 and July 11, 2022, the wavelet multiple correlations showed increasing high levels of correlation through short-to long-terms; with DJI and SP500 dominanting with the tendency to lead or lag in the short-term. The Baruník-Křehlík technique also showed that spillover is higher at short-terms and gradually decreases across the periods. We also report a pair-specific, frequency-dependent connectedness across the assets and indices. Primarily, we show that Non-Fungible Tokens Attention Index (NFTAI) has a higher frequency-based time-varying spillover across assets than CDBC and ICEA. Regulators need to pay close attention to NFTs because they are not fungible and interchangeable neither can their ownership be transferred.

## Highlights

• There is high level connectedness among cross-assets.
• Frequency-dependent spillover is higher is in the short-term.
• Baruník-Křehlík pairwise is pair-specific and frequency dependent.
• Attention indices of digital assets have varying contributions to asset connectedness.
• Non-Fungible Tokens Attention Index (NFTAI) has the highest correlation and causality to other assets; followed by Central Bank Digital Currency Attention Index (CBDCAI) and Index on Cryptocurrency Environmental Attention (ICEA).

## 1 Introduction

Financialisation has contributed to the connectedness of several assets and asset classes such as commodities and financial assets [1]. The degree of connectedness which is frequently characterised by all or most assets moving in a (same) direction, contributes to fluctuations in markets [2]. At different market conditions, with a complex financial system, commodity and financial assets' dependencies tend to vary rather than remain static [3]. For this and other reasons, financial and commodity asset connectedness has been massively studied to inform risk management decisions [4,5]. Among the studies that have explored the connectedness of commodities are [[6], [7], [8], [9], [10]]; financial asset connectedness [[11], [12], [13], [14], [15], [16], [17], [18], [19]]; others have also explored the connectedness of financial and commodity assets – [3,4,[20], [21], [22], [23], [24], [25], [26]]. Another strand of literature has also recorded that assets connectedness increasingly vary during crises [2,6,20,[27], [28], [29],^30^]. The connectedness of assets reportedly increased after the global financial crisis (GFC) in 2006-07 with a sharp magnitude in the markets [6,20,[28], [29], [31], [32], [33], [30]]. With the chaos from the COVID-19 pandemic, another strand of studies sought to explore the pandemic's impact on the connectedness of assets. Studies like [12,[30], [33], [34], [35]] proved that the connectedness of assets showed a series of alterations and spikes, which reflected increased and strong connectedness due impacts from the pandemic. These reflect how crises can distract and cause alterations in asset connectedness.

The article "Connectedness in cross-assets and digital assets attention indices" was published in 2023. Journal: Heliyon.

Since financialisation's contribution to asset connectedness mostly after the GFC [20,[36], [37], [38], [39]], other digital assets have also gained investor interest. In more recent times, digital assets such as Decentralised Finance (Defi), Cryptocurrency, and Non-Fungible Tokens (NFT) are investment avenues used to detach from risk. The rise in the usage of cryptocurrencies during the COVID-19 pandemic only re-enforces the main aim of decentralising finance from the government and the fact that individuals are wrestling economic and financial power from the national and international governments [13,15,40,41]. On the other hand, the progress in peer-to-peer transactions as well as huge investments in digital currencies and their associated novel assets should be of concern to any responsible central government because that is a sign of deversion of financial resources from other sectors of the economy, such as banking, manufacturing, bonds, stocks, among others. For instance, cryptocurrencies (i.e. Bitcoin) has been referred to as the new gold and hence serves as a diversifier, hedge, and safe haven [42,43]. One could argue that the frenzy by central governments to adopt digital currencies as Central Bank Digital Currencies (CBDCs) point to the potential and the already desirable features of digital currencies and assets. Is not surprising that there is has been a natural feedback loop between these unconventional assest and well-known financial assets and commodities. It is worth nothing that despite the fuss about digital currencies, the risks in these are also quite pronounced as revealed in their high levels of volatilies and episodic market crushes [17,44]. This has created a competition over financial and economic resources needed for both risk management and reward seeking investors as well as concern for policy-makers.

The article "Connectedness in cross-assets and digital assets attention indices" was published in 2023. Journal: Heliyon.

Hence, the relationship between digital currencies and assets has been the focus of many a spillover, connectedness, interdependence, comovement, and information transfer studies in the recent literature [40,41,45,46]. Some studies that have contributed to the connectedness of conventional assets and digital assets are [19,22,24,47,48], reporting varying spillover effects. It is said that NFTs and Defi are decoupled from other assets due to the asymmetry of information in these markets [17,19,49,50]. During the recent pandemic [51], found that digital assets such as NFTs were primarily independent of shocks transmitted from other markets and cryptocurrencies [47]. The pricing of NFTs as in Ref. [47] showed that though decoupled from other assets, is partly dependent on transmissions from cryptocurrency prices. With the benefits of speculative investments in the cryptocurrency markets [52,53] and its transmission to NFT pricing, how does the popularisation of NFTs affect other assets’ connectedness? Also, we use the Central Bank Digital Currency attention index (CBDCAI) because the growing risk from these digital assets could be easily transferred to banks and financial institutions due to the nature of the financial system [54]. [55] also found an interdependent relationship between Central Bank Digital Currency (CBDC) and stock markets and noted that the strong correlation is based on the CBDC attention index. The CBDCs, although, have not been adopted by countries yet, news about such centralised government securities that intend to promote the financial security of banks could have impacts on asset connectedness. Also, with growing and interest in cryptocurrencies, we use the Index on Cryptocurrency Environmental Attention (ICEA) to capture the environmental attention on cryptocurrencies to the connectedness of assets. The continuous mining of digital assets based on distributed ledger technology and electricity usage result in greenhouse gas (GHG) emissions which may have impacts on assets especially green stocks [56]. showed how green stocks can be used as diversifiers for Bitcoin and in commodity markets (except precious metals) [21]. If so, and the GHG emissions are increasing based on increasing volumes of cryptocurrency mining [57], how does the ICEA affect connectedness in assets since investors would want to move to green-based assets**.** Also, the increased connectedness of conventional assets raises alarm for significant interdependent risk in the markets. Thus, if there is increased attention from cryptocurrency mining as the ICEA captures, what would be its effect on the connectedness of cross-assets. Aside from Ref. [50] who explored the connectedness of the NFT index on other financial markets, no literature according to our knowledge has explored how financial and commodity asset connectedness has changed prior to the emergence of digital assets (Defi, Cryptocurrency, and NFT) and its financialisation. Thus, using the wavelet technique, we examine the connectedness of 12 cross-assets (if any), and use the frequency spillover of [58] to explore how the connectedness is altered following the advent of digital assets using respective attention indices. We are interested in using the attention indices because digital assets are continually contributing to investor needs for hedging, diversification, safe-haven, and as a store of value.

The article "Connectedness in cross-assets and digital assets attention indices" was published in 2023. Journal: Heliyon.

Thus, we first explore the connectedness of assets from energy, agricultural commodities, precious metals, and some stock indices using the wavelet multiple correlation analysis. We further explore the connectedness, if any, of these financialised assets as and when digital assets were settling in the minds of investors using [58]'s (Baruník-Křehlík) frequency domain spillover index. In order to fully capture the frequency dynamics of connectedness [25], we decompose the connectedness into bands that correspond to short-, medium-, and long-terms (as frequencies) suiting different preferences of economic agents. The extant literature supports the notion that economic agents work at different investment horizons pursuant to their risk and return preferences [[59], [60], [61], [62]]. One of the main advantages of the frequency-domain techniques over other methods to study connectedness is the ability to enable a multi-scale analysis of time series in frequencies [5]. We employ the wavelet multiple correlation (WMC), wavelet multiple cross correlation (WMCC) and Baruník-Křehlík techniques in this paper.

The findings from the WMC and WMCC show high correlations among the assets with SP500 and DJI dominating in the short-term with the tendency to lead or lag and Silver lagging in the long-term. With the observed high level of correlation, when we further incorporated the attention indices, we found that the spillovers (static and rolling) are driven by short-horizons dynamics and the market is more responsive in the short-term. In line with the efficient market hypothesis [63], investors respond quickly to information in the market and on assets based on the heterogeneity of preferences for risk as in the competitive market hypothesis [64]. In the long-term, however, connectedness is persistent and transmitted gradually based on investor adaptiveness to the efficiency in the market [65]. The spillover indices were higher at higher frequencies and reduced across the bands based on the adaptive and heterogenous nature of investors in the markets [65,66]. The static and rolling pairwise net spillovers were unique to the pair and frequency of the analysis. Thus we report a pair-specific and frequency-dependent connectedness in the conventional assets and digital assets. Lastly, we found that the spillover is higher for the assets and NFT attention index (NFTAI) than CBDCAI and the least spillover is when ICEA is introduced to assets’ connectedness. Theoretically, this shows how investors respond to the dynamics in the markets in the short-term.

The article "Connectedness in cross-assets and digital assets attention indices" was published in 2023. Journal: Heliyon.

Cross-assets are highly connected in developed and liquid markets showing how homogeneous and competitive the markets are [17,18,[26], [27], [28],^32^,^30^]. In the short-term however, investors are more responsive to news in the market which reflects immediately in asset prices as compared to the medium- and long-term [15,63]. Thus, in such efficient and highly connected markets, investors should look out for hedging benefits as compared to diversification benefits [6,9,15]. This is because of the level of exposure in these markets which lead to increased exposure to interdependent risk. We have shown that there is high connectedness between cross-assets and how such connectedness fluctuates when attention indices of digital assets are introduced. Though investors are moving to digital assets, we have showed that CBCDs can provide hedging benefits to cross-assets because of its centralised and controlled effects because it shows less correlation and causality to the cross-assets. At different horizons, investors can coup from ICEA but that depends on the sentiments investors may have on the level of mining and the effect it may have on the environment. Irrespective, there is no dominance in ICEA's ability to lead the prices of cross-asset markets. Investors are however cautioned on NFTs as it is gaining more attention in the markets and has the highest correlation among the other digital assets attention indices. It is important for investors in NFTs to note that risks in that market are still evolving and thus, it is important for thorough research before engaging in NFT investments.

The rest of the paper is in sections; methods, data and preliminary analysis, results and analysis, and the conclusions.

## 2 Methods

### 2.1 WMC and WMCC

Let the data generation process be represented by a multivariate stochastic process ($Z_{t}=z_{1t},z_{2t},\ldots ,z_{nt}$) and the accompanying scale $\vartheta_{j}$ be represented by ($W_{jt}=w_{1jt,}w_{2jt},\ldots ,w_{njt}$). Then, each $z_{it}$ is subjected to the maximal overlap discrete wavelet transform (MODWT) to produce wavelet coefficients. The MODWT is applied to each of the weekly variables and indices returns as indicated by Ref. [67] in order to calculate WMC and WMCC. The WMC, denoted by $C_{Z}\left(\vartheta_{j}\right)$ is a single set of multivariate scale correlations as [68];

(1) $$C_{Z}\left(\vartheta_{j}\right)={\left(1-\frac{1}{\max\;diagP_{j}^{-1}}\right)}^{0.5}$$

For each $\vartheta_{j}$, the linear combination of $w_{ijt},i=1,2,\ldots ,n$ is used to compute the square roots of the coefficient of determination of the regression ($R^{2}$) for which a maximum value for $R^{2}$ is determined. A coefficient of determination can be obtained from a regression of a regressand $y_{i}$ on a set of predictors {$y_{k},k\neq i$}, as Ri2=1−1ρii, $i^{th}$ diagonal element of the inverse of the complete correlation matrix P. $P_{j}$ is the q×q correlation matrix of $W_{jt}$ and maxdiag(*) elects the maximum element in the diagonal argument.

The article "Connectedness in cross-assets and digital assets attention indices" was published in 2023. Journal: Heliyon.

Following the theory of regression, we finally define WMC as [68,69];

(2) $$C_{Z}\left(\vartheta_{j}\right)=\frac{Corr\left(w_{i\;jt},{\hat{w}}_{i\;jt}\right)Cov\left(w_{i\;jt},{\hat{w}}_{i\;jt}\right)}{\sqrt{Var\left(w_{i\;jt}\right)Var\left({\hat{w}}_{i\;jt}\right)}}\text{,}$$

where $w_{ij}$ is chosen to maximise $C_{Z}\left(\vartheta_{j}\right)$ and ${\hat{w}}_{i\;jt}$ are the fitted values in the regression of $w_{ij}$ on the rest of the wavelet coefficients at $\vartheta_{j}$.

The WMCC is also set as below, allowing a lag (τ) between the observed ($y_{i}$) and fitted values (${\hat{y}}_{i}$) at each $\vartheta_{j}$ as [[67], [68], [69]]:

(3) $$C_{Z},\tau \;\left(\vartheta_{j}\right)=Corr\left(w_{i\;jt},{\hat{w}}_{i\;jt+\tau }\right)=\frac{Cov\left(w_{i\;jt},{\hat{w}}_{i\;jt+\tau }\right)}{\sqrt{Var\left(w_{i\;jt}\right)Var\left({\hat{w}}_{i\;jt+\tau }\right)}}$$

we chose to use J=6 for shape parameters [68]. The number of feasible wavelet coefficients gets critically small for high levels thus a scale J>6 is not advisable. Each J produces J number of wavelet coefficients and J−(J−1) scaling coefficient [[67], [68], [69]].

### 2.2 Frequency domain spillover index

Using a matrix of decomposed vector autoregressive (VAR) based on generalised forecast error variance decompositions (GFEVD), we measure the connectedness of the variables in this study on a frequency domain approach [65]. For the matrix of decomposed VAR, we consider a stationary covariance with a *Z*-variate process $K_{t}={\left(k_{1,t},\ldots ,k_{Z,t}\right)}^{\prime }$ at t=1,…,T and VAR of order φ is also [9,58];

(4) $$K_{t}=\sum_{i=1}^{\varphi }\psi_{i}k_{t-i}+\epsilon_{t}$$

where $\psi_{i}$ and $\epsilon_{t}$ are coefficient matrices and noise with (likely non-diagonal) covariance matrix φ. Each variable is regressed on its lags (φ) and of all the other variables. ψ contains all the information on the connectedness between the variables. Note the usefulness of working with a (Y×Y) matrix $\left(I_{Y}-\prod_{1}L-\ldots -\prod_{\varphi }L^{\varphi }\right)$ with identity $I_{Y}$. If the roots of the characteristic equation |θ(z)| lie outside of the unit circle, the VAR system has a moving average MA(∞) [58]:

(5) $$Y_{t}=\emptyset \left(L\right)\epsilon_{t}$$

with ψ(L) being an infinitely lagged polynomial. The GFEVD which is the contribution of the yth variable to the variance of forecast error of the element j can be written as [9,16,58]:

(6) $${\left(\Theta_{Q}\right)}_{j,y}=\frac{\sigma_{yy}^{-1}\sum_{q=0}^{Q}{\left({\left(\psi_{q}\varphi \right)}_{j,y}\right)}^{2}}{\sum_{q=0}^{Q}{\left(\psi_{q}\varphi_{q^{\prime }}\right)}_{j,y}}$$

where q=1,…,H and $\sigma_{yy}=\left(\varphi_{yy}\right)$. The transformations of $\emptyset_{q}$ serve as a contribution to the shocks of the system for which the decomposed connectedness measure is possible. Since the sum of the contributions in the row is not one, the matrix $\Theta_{Q}$ is further standardised as [16,58];

(7) $${\left({\tilde{\Theta }}_{Q}\right)}_{j,y}=\frac{{\left(\Theta_{Q}\right)}_{j,y}}{\sum_{k=1}^{N}{\left(\Theta_{Q}\right)}_{j,y}}$$

From equation (7), the total and pairwise connectedness can be computed. According to Ref. [70], the connectedness can be defined as the share of variance in the forecasts contributed by errors other than their own error (or the ratio of the sum of the off-diagonal elements to the sum of the entire matrix) as in Refs. [16,70,71];

(8) $$C_{Q}=100*\frac{\sum_{j\neq y}{\left({\tilde{\Theta }}_{Q}\right)}_{j,y}}{\sum {\tilde{\Theta }}_{Q}}=100*\left(1-\frac{\Omega r\left\{{\tilde{\Theta }}_{Q}\right\}}{\sum {\tilde{\Theta }}_{Q}}\right)$$

where Ωr{.} is the trace operator, the denominator is the sum of all elements in the matrix. Now, it is apparent that the connectedness shows the relative contribution of the forecast variance from the other variables in the system and hence bi-directional (“*to”* variable *m* from all other variables n, and vice versa (“*from”*)) connectedness. Also, “*net”* connectedness is measured as the difference between “*to”* and “*from”* spillovers – a variable with a positive (negative) net spillover is a net transmitter (recipient) of shocks.

The article "Connectedness in cross-assets and digital assets attention indices" was published in 2023. Journal: Heliyon.

At this stage, the spectral representation of connectedness is presented. Given a frequency response function of $\emptyset {\left(e\right)}^{-i\omega }=\sum_{q}e^{-i\omega h}\emptyset_{q}$ of Fourier transformable coefficients $\emptyset_{q}$ with $i=\sqrt{-1}$, a spectral density of $Y_{t}$ at frequency ω can be defined as MA(∞) filtered series [16,58];

(9) $$S_{y\left(\omega \right)}=\sum_{h=-\infty }^{\infty }E\left(Z^{\prime }Z_{t-q}\right)e^{-i\omega q}=\emptyset {(e}^{-i\omega })\varphi \emptyset^{\prime }{(e}^{+i\omega })$$

The power spectrum $S_{y\left(\omega \right)}$ describes the distribution of the variance of $Y_{t}$ over the frequency components ω. The causation spectrum over ω∈(−π,π) presents the portion of the mth variable due to shocks in the nth variable at a given frequency ω. It follows that [16,58];

(10) $${\left(F\left(\omega \right)\right)}_{j,y}=\frac{\sigma_{yy}^{-1}{{\left(\emptyset {(e}^{-i\omega }\right)\varphi }_{j,y})}^{2}}{{\left(\emptyset {(e}^{-i\omega }\right)\varphi \emptyset^{\prime }{(e}^{+i\omega }))}_{j,j}}$$

can be interpreted as *within-frequency* causation on account of the denominator. It is only regular to weight ${\left(F\left(\omega \right)\right)}_{j,y}$ by the frequency share of the variance of the jth variable in order to obtain a natural decomposition of GFEVD to frequencies. The weighting function can be defined as [16,58];

(11) $$\Gamma_{j}=\frac{{\left(\emptyset {(e}^{-i\omega }\right)\varphi \emptyset^{\prime }{(e}^{+i\omega }))}_{j,j}}{\frac{1}{2\pi }\int_{-\pi }^{\pi }{\left(\emptyset {(e}^{-i\gamma }\right)\varphi \emptyset^{\prime }{(e}^{+i\gamma }))}_{j,j}d\gamma }$$

summing up real-valued numbers up to 2π and denotes the power of the jth variable at a given frequency. Practical financial applications require measuring connectedness over time horizons. Hence, it is appropriate to quantify connectedness over frequency bands rather than at single frequencies. In formal terms, for a frequency band d=(a,b):a,b∈(−π,π),a<b, the GFEVDs is [9,16,58];

(12) $${\left(\Theta_{d}\right)}_{j,k}=\frac{1}{2\pi }\int_{a}^{b}{\Gamma_{j}\left(\omega \right)\left(F\left(\omega \right)\right)}_{j,y}d\omega \text{.}$$

Over the same frequency band d, a scaled generalised variance decomposition can be defined in Refs. [57,71,72];

(13) $${\left({\tilde{\Theta }}_{d}\right)}_{j,k}={\left(\Theta_{d}\right)}_{j,k}/\sum_{k}{\left(\Theta_{\infty }\right)}_{j,k}\text{.}$$

Subsequently, the *within-frequency* and frequency connectedness over d are defined in equations (14), (15), respectively [57,58,71,72];

(14) $$C_{d}^{W}=100.\left(1-\frac{\Omega r\left\{{\tilde{\Theta }}_{d}\right\}}{\sum {\tilde{\Theta }}_{d}}\right)$$

(15) $$C_{d}^{F}=100.\left(\frac{\sum {\tilde{\Theta }}_{d}}{\sum {\tilde{\Theta }}_{\infty }}-\frac{\Omega r\left\{{\tilde{\Theta }}_{d}\right\}}{\sum {\tilde{\Theta }}_{\infty }}\right)=C_{d}^{W}.\left(\frac{\sum {\tilde{\Theta }}_{d}}{\sum {\tilde{\Theta }}_{\infty }}\right)$$

$C_{d}^{W}$ shows the connectedness within a frequency band and it is weighted exclusively by the power of the series on the given frequency band. Yet, $C_{d}^{F}$, decomposes the overall connectedness into discrete parts which sum up to the original connectedness measure [58]. We use the frequency bands (″π+0.00001,π/4,π/24,0″) [57,71,72].

The article "Connectedness in cross-assets and digital assets attention indices" was published in 2023. Journal: Heliyon.

## 3 Data and preliminary analysis

In this study, we employ weekly frequency of the data series. This is informed on the fact that the digital asset attention indices are only reported in weekly frequencies. While the other conventional assets come in various periodicities, we collect them in weekly frequencies to ensure uniformity and to foster comparison. The financial assets (Dow Jones Industrial Average (DJI), FTSE 100 (FTSE), Nikkei 225 (Nikkei) and S&P 500 (SP500)) and commodity assets (Coffee, Cotton), energy (Crude oil, Natural Gas) and metals (Gold, Palladium, Platinum, Silver) were downloaded using the yfR package in R (https://cran.r-project.org/web/packages/yfR/index.html). We opted to capture each sector of interest to investors and have continually been proven to show connectedness. To explore if the theorised financial and commodity connectedness is disrupted when digital assets are included, we use the weekly attention indices of NFTs, CBDC and cryptocurrency environmental attention (CEA) extracted from https://sites.google.com/view/cryptocurrency-indices/home?authuser=0. The ICEA to some broader extent has relationships with the most capitalised cryptocurrency (Bitcoin), cryptocurrency uncertainty indices and captures major events that cause fluctuations in prices of digital assets (see Ref. [73]). Thus, using the ICEA, we would be able to determine (if any) the impacts of CEA on other assets. Financial markets are sensitive to CBDCAI and have a significant negative relationship [74]. Thus, we sought to explore how this sensitivity disrupts asset connectivity. We also use NFTAI because literature has proven that NFT is decoupled from other assets but has a fair market capitalisation compared to other digital assets [https://coinmarketcap.com/view/collectibles-nfts/] ([50]).

We used returns computed as $r_{t}=\ln\;P_{t}-\ln\;P_{t-1}$ for each variable; $r_{t}$ (continuously compounded returns), $P_{t}$ (current variable price), $P_{t-1}$ (previous variable price). The financial and commodity assets were sampled from 25 January 2010 to 11 July 2022 with 467 observations and expressed in USD. The indices, however, have varying observations as shown in Table 1 as and when the data were available (CBDCAI – 09 January 2015 to 29 April 2022; ICEA – 10 January 2014 to 29 April 2022; NFTAI – 20 January 2017 to 29 April 2022). The data shows non-normality at 1 %, presence of kurtosis and negative (positive) skewness mostly for the financial and commodity assets (digital asset attention indices). The mean of all the distributions is positive except for Platinum. The graphical representation of the assets is in Fig. 1 – reflecting volatility.

The article "Connectedness in cross-assets and digital assets attention indices" was published in 2023. Journal: Heliyon.

**Table 1:** Descriptive statistics.

	Mean	Std. Dev.	Skewness	Kurtosis	Normtest W.	ADF	KPSS	Obs.
Financial Assets								
Coffee	0.0007	0.0503	0.2258	1.5719	0.9842***	−7.2000***	0.1300	467
Cotton	0.0006	0.0522	−2.0341	17.4608	0.8507***	−6.2000***	0.0680	467
Crude Oil	0.0004	0.0642	−0.1238	7.0647	0.9092***	−9.0000***	0.0970	467
Natural Gas	0.0004	0.0753	−0.0431	1.5146	0.9829***	−8.0000***	0.2600	467
Gold	0.0009	0.0252	−0.2646	1.7241	0.9791***	−7.5000***	0.1100	467
Palladium	0.0031	0.0589	−0.7941	11.5213	0.8994***	−8.6000***	0.0700	467
Platinum	−0.0013	0.0396	−0.2972	3.2976	0.9590***	−9.9000***	0.0390	467
Silver	0.0000	0.0489	−0.7648	5.7940	0.9323***	−8.1000***	0.0880	467
DJI	0.0023	0.0274	−0.8936	7.8988	0.9070***	−9.9000***	0.0330	467
FTSE	0.0006	0.0262	−1.2441	7.5091	0.9187***	−10.0000***	0.0300	467
Nikkei	0.0019	0.0338	−0.4671	3.5908	0.9540***	−7.9000***	0.0550	467
SP500	0.0026	0.0274	−0.8638	5.0392	0.9256***	−9.8000***	0.0320	467
**Attention Indices**								
CBDCAI	0.0001	0.006	1.4745	17.0358	0.6633***	−8.0000***	0.0350	274
ICEA	0.0001	0.0047	3.3873	50.6822	0.5809***	−9.1000***	0.1000	313
NFTAI	0.0002	0.0060	1.1458	63.3766	0.3599***	−8.8000***	0.1400	197

Note: (***) denote significance at 1 %. Obs. (Observation), Std. Dev. (Standard Deviation).

**Fig. 1:** Prices (Panel A) and returns (Panel B) of cross-assets and digital assets attentition indices.

## 4 Results and discussion

The data analysis is in four sections. We first check for the connectedness of the financial and commodity assets using the wavelet technique. At lag 6, the scales for the WMC and WMCC are $w_{i1}:2∼4$ (month), $w_{i2}:4∼16$ (month to semi-annual) and $w_{i3}:16$ *∼*32 (semi-annual to annual). We further use the Baruník-Křehlík technique to find the frequency spillover effect on the assets’ connectedness when the digital assets attention indices are introduced. Setting the lag at 1, for each index, we examine the alterations in the connectedness. The bands for the frequency domain spillover are $d_{1}:3.14∼0.79$ (month), $d_{2}:0.79∼0.13$ (month to semi-annual) and $d_{3}:0.13∼0.00$ (semi-annual to infinity).

The article "Connectedness in cross-assets and digital assets attention indices" was published in 2023. Journal: Heliyon.

### 4.1 WMC and WMCC analysis

The WMC outputs are presented in Table 2 (Panel A) and Fig. 2. The outputs show the degree of connectedness among the respective financial and commodity assets’ returns. From Fig. 2, the degree of connectedness as measured by correlation (as in Table 2), show that the assets are highly correlated. In Table 2 (Panel A), the WMCs are generally increasing throughout the period. This means that there is high integration between the assets increases from the short-term to the long-term. The degree of integration for the weekly return series is comparatively high at 0.962795 for scale 1 and 0.9999 for WMC at scale 32.

**Table 2:** Wavelet multiple correlations and cross-correlations.

Panel A				Panle B		
Scale	WMC ‘lower’	Correlation	WMC ‘upper’	Localisation	Time Lag	Leading/Lagging variables
	WMC			WMCC		
1	0.962795	0.971147	0.977645	0.971147	0	DJI
2	0.967634	0.977504	0.984387	0.977504	0	SP500
4	0.969122	0.981683	0.989162	0.981683	0	DJI
8	0.978371	0.989915	0.995312	0.989915	0	SP500
16	0.948521	0.983925	0.995042	0.983925	0	Platinum
32	0.999958	0.999994	0.999999	0.999997	12.5	Silver

Note: The upper and lower columns are at 5 % significant levels presenting the high correlations of the cross-assets.

**Fig. 2:** WMC of 12 cross-assets (financial and commodity assets).

The WMCC (Panel B of Table 2) outputs help to identify which of the assets is leading (negative localisation) or lagging (positive localisation) or can lead or lag (at localisation 0). A dominant asset across the scales may pose contagion effects to other markets and at scales where there is no dominance, the assets are reported to be interdependent of each other. These inform investors’ diversification and safe-haven decisions. In Fig. 3, we show that DJI and SP500 are interchangeably dominant among other assets and also have the tendency to lead or lag the other assets just as Platinum too at localisation 0. Silver, however, in the long run, is the lagging asset at 12.5.

**Fig. 3:** WMCC of 12 cross-assets, *Note: Localisations are the boldened dashed-lines*.

While we expect to integrate in the long-term, even for unrelated assets [68], to erode the benefits of diversification, it is surprising to see that these assets are strongly correlated (especially so of assets of different classes) from the short-term (from the weekly – wavelet scale 1 to the monthly (wavelet scale 4)) through to the long-term (from quarterly wavelet scale 16 to semi-annually – wavelet scale 32). Nonetheless, a deeper look from Fig. 3 reveals that this can be a result of financialisation of the commodities markets, as with many other markets [3,4,[20], [21], [22], [23],^23^,^25^,[26], [75]]. Due to this, it has become more and more difficult to distinguish between assets as the boundaries have become fuzzy due to their technological drive and price generating processes.

The article "Connectedness in cross-assets and digital assets attention indices" was published in 2023. Journal: Heliyon.

In addition, the high correlations recorded also imply that these assets are affected by similar news on market shocks; partly by market cycles; financial interdependencies and, are driven mostly by the same macroecnomic and financial variables [[76], [77]]. Because of this high correlation among the assets, the benefit from diversification are almost non-existent even in the short-term [75,78,79] but hedging is necessary to avoid extreme losses in the markets if any in the long-term [80].

Generally, highly correlated assets increase the risk exposure of a portfolio due to the contribution from the market and the volatility in prices. It would rather be better for investors who may want to diversify to benefit from market transparency through risk disclosures and pricing mechanisms for such high correlated assets. However, because of the efficiency in the markets and investor behavioural tendencies, prices cannot be expansively regulated. However, policy-makers can adapt regulations and policies to address the risk in the markets by protecting investor interests. Investors may also hedge against any excessive losses that they may experience in the markets especially in the short-term.

### 4.2 Frequency-time domain connectedness analysis

We use the Baruník-Křehlík connectedness technique to explore whether the asset connectedness alters over time as and when the attention indices were introduced. We present the static (as in tables) and rolling over (as in graphs) spillover connectedness of the respective indices and the assets. In the tables for total and net spillovers, the absolute (ABS) and within (WTH) spillover indices are boldened and italised. The highest spillover index from the variables is in bold. WTH connectedness measures causality rather than correlation which is ABS connectedness.

From Table 3, at the bands, we observe a reducing spillover across the bands. A reducing spillover across bands show how investors’ activities at different frequencies alter the connectedness of variables [58]. Theoretically, investors in the markets are more efficient in the short-term as compared to the medium- and long-terms especially for developed and liquid markets. In such markets, investors are more responsive to news and shocks which is immediately reflected in assets prices. At Band 1, the level of spillover is high and this attributably, maybe a result of calm and accurate investor behaviour in reacting to information in the markets [58,63]. Comparatively, we show that the spillover across bands 2 and 3 gradually reduce in line with [16,71] who also show that, at higher frequencies, connectedness increases [58]. conclusively also confirm that persistently, at lower frequencies, shocks are transmitted over time which allows investors to heterogeneously adapt to the markets [65,66]. We report a decreasing return spillover from 38.36 (Band 1), 8.14 (Band 2) to 2.06 (Band 3). Our results show that investors are more responsive to the market in the short-term as compared to the longer-term. With the level of high correlations as shown in the wavelet results, this results was expected. The cross-assets used in this study are in developed markets and liquid implying a homogeneous competitive market in the short-term than in the long-term; as investors may eventually adapt in the market and diversify away risk. Also, in the long-term, investors in the market become more heterogenous to risk preferences and needs which provides a less risky investment market – thus, the reduced spillover effects. The net spillover also shows a reducing spillover across the bands. We show that averagely, Coffee, Natural gas, Palladium, Platinum, Silver, DJI, FTSE and SP500 are net transmitters in the spillover network while CBDCAI, Cotton, Crude oil, Gold and Nikkei are net receivers across bands with decreasing spillover effects. Across the bands, we find that averagely, precious metals and stock indices are dominant in leading the prices of agricultural commodities. In a highly correlated cross-assets as has been shown precious metals could be used as safe-haven making it more susceptible to investors desire to diversify against risk in a portfolio [15,81]. Also, in developed stock markets, there is a high level of liquidity and efficiency. As such, they incorporate information into their prices fast due to the presence of sophisticated market participants and wide range of financial instruments and services, hence, its ability to dominate the markets. Because of the level of responsiveness in developed stock markets [82], found that emerging markets are more suitable to provide hedging benefits for commodities.

The article "Connectedness in cross-assets and digital assets attention indices" was published in 2023. Journal: Heliyon.

**Table 3:** Total and net spillover indices between the assets and CBDCAI.

	Coffee	Cotton	Crude Oil	Natural Gas	Gold	Palladium	Platinum	Silver	DJI	FTSE	Nikkei	SP500	CBDCAI	FROM_ABS^a^	FROM_WTH^b^
*Band 1: 3.14 to 0.79; corresponds to 1 to 4 Weeks*															
Coffee	69.28	2.03	0.39	1.17	2.07	1.81	2.35	2.93	0.92	0.41	0.18	0.93	0.43	1.20	1.50
Cotton	0.63	50.18	1.87	1.65	0.29	0.48	2.05	0.57	5.41	3.21	2.17	5.47	0.21	1.85	2.30
Crude Oil	0.53	1.28	37.57	1.07	0.38	2.80	4.33	3.32	5.12	5.75	2.9	4.91	0.22	2.51	3.13
Natural Gas	1.49	2.12	0.81	71.89	0.37	0.57	0.16	0.02	1.76	0.04	0.59	2.01	0.12	0.77	0.96
Gold	1.75	0.24	0.20	0.22	36.38	7.52	11.91	22.25	0.15	0.39	0.53	0.18	0.14	3.5	4.36
Palladium	0.14	0.57	2.15	0.58	7.93	38.03	11.77	10.62	3.52	2.95	1.98	2.6	0.45	3.48	4.34
Platinum	0.44	1.23	2.56	0.82	9.28	9.40	30.17	12.88	3.82	3.56	1.45	3.18	0.23	3.76	4.68
Silver	1.01	0.29	2.38	0.01	18.05	8.15	13.01	29.89	2.75	1.61	0.32	2.66	0.28	3.89	4.84
DJI	0.12	2.85	2.86	2.03	0.26	2.19	2.85	1.95	22.75	11.26	10.20	21.26	0.08	**4.45**	**5.55**
FTSE	0.32	1.62	3.99	0.58	0.10	2.39	2.99	1.28	14.95	26.6	11.77	13.78	0.27	4.16	5.18
Nikkei	0.28	0.94	1.85	0.99	0.70	2.00	1.98	0.60	13.95	12.23	29.94	13.48	0.07	3.77	4.70
SP500	0.17	2.80	2.84	2.22	0.23	1.66	2.52	1.96	22.1	10.84	10.44	23.48	0.06	**4.45**	5.54
CBDCAI	0.93	0.93	0.55	0.75	0.29	0.51	0.59	0.35	0.2	2.13	0.09	0.12	78.36	0.57	0.71
TO_ABS^a^	0.60	1.30	1.73	0.93	3.07	3.04	4.35	4.52	5.74	4.18	3.28	5.43	0.2	***38.36***	
TO_WTH^b^	0.75	1.62	2.15	1.16	3.83	3.79	5.42	5.63	7.16	5.21	4.09	6.77	0.24		***47.80***
Net	−0.60	−0.56	−0.78	0.16	−0.43	−0.45	0.59	0.63	1.29	0.03	−0.50	0.98	−0.38		
*Band 2: 0.79 to 0.13; corresponds to 4 to 24 Weeks*															
Coffee	11.20	0.02	0.17	0.21	0.05	0.19	0.01	0.06	0.03	0.00	0.04	0.02	0.16	0.07	0.46
Cotton	0.12	10.64	1.20	0.55	0.02	0.08	0.61	0.23	1.95	1.81	1.12	2.16	0.01	0.76	4.80
Crude Oil	0.01	0.16	11.44	0.02	0.10	1.18	2.01	1.05	1.58	2.91	1.55	1.55	0.09	0.94	***5.95***
Natural Gas	0.09	0.89	0.25	11.61	0.23	0.02	0.04	0.00	0.39	0.02	0.34	0.5	0.04	0.22	1.37
Gold	0.66	0.16	0.05	0.03	6.88	1.07	1.70	3.79	0.01	0.02	0.18	0.01	0.03	0.59	3.75
Palladium	0.02	0.02	0.31	0.12	1.01	6.8	1.80	1.40	0.44	0.80	0.39	0.31	0.02	0.51	3.23
Platinum	0.17	0.37	1.02	0.01	1.90	1.57	5.41	2.64	0.81	1.58	0.52	0.74	0.01	0.87	5.53
Silver	0.37	0.01	0.95	0.01	3.31	1.30	2.48	5.62	0.43	0.64	0.10	0.46	0.02	0.77	4.91
DJI	0.00	0.31	0.87	0.02	0.03	0.57	0.61	0.49	3.73	3.31	1.99	3.54	0.01	0.90	5.72
FTSE	0.01	0.28	1.16	0.06	0.01	0.29	0.42	0.22	2.53	5.97	1.99	2.49	0.02	0.73	4.62
Nikkei	0.16	0.34	0.59	0.00	0.34	0.14	0.10	0.01	2.67	3.74	5.8	2.84	0.01	0.84	5.33
SP500	0.00	0.38	0.76	0.01	0.03	0.38	0.50	0.47	3.55	3.07	1.96	3.84	0.01	0.86	5.42
CBDCAI	0.21	0.05	0.05	0.19	0.07	0.21	0.04	0.10	0.02	0.02	0.01	0.03	0.39	**10.08**	0.48
TO_ABS^a^	0.14	0.23	0.57	0.09	0.55	0.54	0.79	0.81	1.11	1.38	0.78	1.13	0.03	***8.14***	
TO_WTH^b^	0.89	1.45	3.60	0.60	3.46	3.40	5.03	5.11	7.02	8.73	4.96	7.13	0.20		***51.58***
Net	0.07	−0.53	−0.37	−0.12	−0.05	0.03	−0.08	0.03	0.20	0.65	−0.06	0.27	−0.04		
*Band 3: 0.13 to 0.00; corresponds to infinite weeks*															
Coffee	2.74	0.00	0.05	0.05	0.01	0.04	0.00	0.01	0.00	0.00	0.01	0.00	0.04	0.02	0.42
Cotton	0.03	2.71	0.33	0.14	0.00	0.02	0.16	0.06	0.51	0.49	0.30	0.57	0.00	0.20	5.07
Crude Oil	0.00	0.05	2.97	0.00	0.02	0.30	0.53	0.27	0.42	0.78	0.41	0.41	0.02	**0.25**	**6.22**
Natural Gas	0.02	0.24	0.07	2.88	0.06	0.00	0.01	0.00	0.10	0.01	0.09	0.13	0.01	0.06	1.44
Gold	0.17	0.04	0.01	0.01	1.69	0.25	0.41	0.92	0.00	0.00	0.05	0.00	0.01	0.14	3.62
Palladium	0.01	0.00	0.07	0.03	0.24	1.66	0.44	0.33	0.1	0.20	0.09	0.07	0.00	0.12	3.08
Platinum	0.04	0.10	0.27	0.00	0.47	0.37	1.35	0.66	0.21	0.41	0.14	0.19	0.00	0.22	5.55
Silver	0.09	0.00	0.25	0.00	0.81	0.31	0.62	1.39	0.11	0.17	0.03	0.12	0.00	0.19	4.87
DJI	0.00	0.08	0.22	0.00	0.01	0.14	0.15	0.12	0.92	0.84	0.49	0.88	0.00	0.23	5.70
FTSE	0.00	0.07	0.30	0.01	0.00	0.07	0.11	0.06	0.64	1.51	0.50	0.63	0.00	0.18	4.65
Nikkei	0.04	0.09	0.15	0.00	0.09	0.03	0.03	0.00	0.68	0.96	1.45	0.73	0.00	0.22	5.43
SP500	0.00	0.09	0.19	0.00	0.01	0.09	0.13	0.12	0.88	0.77	0.48	0.95	0.00	0.21	5.38
CBDCAI	0.05	0.01	0.02	0.05	0.02	0.05	0.01	0.03	0.00	0.00	0.00	0.01	2.56	0.02	0.47
TO_ABS^a^	0.03	0.06	0.15	0.02	0.13	0.13	0.20	0.20	0.28	0.36	0.20	0.29	0.01	***2.06***	
TO_WTH^b^	0.86	1.50	3.76	0.57	3.36	3.28	5.02	5.02	7.09	8.96	5.02	7.25	0.20		***51.89***
Net	0.02	−0.14	−0.10	−0.03	−0.01	0.01	−0.02	0.01	0.06	0.17	−0.02	0.07	−0.01		

Note.

a Absolute to measures return spillovers from asset m to other assets. Absolute from measures return spillovers from other assets to asset m.

b Within to measures return spillovers from asset m to other assets, including from own innovations to asset n. Within from measures return spillovers from other assets to asset m, including from own innovations to asset n [71,83]. The largest contributions of assets per frequency band are in bold italics. Positive **Net** denotes that the asset is a **net transmitter** [an asset that can dominate and cause systemic risk; lead the price fluctuations in other assets] while negative **Net** denote **net recipient** [an asset that is less dominant and more vulnerable to external shocks].

The article "Connectedness in cross-assets and digital assets attention indices" was published in 2023. Journal: Heliyon.

Because we want to explore how the integration or the attention of digital assets alters assets connectedness, we further take a look at the spillover to and from the assets to CBDCAI. In this connectedness, we observe here again that the spillover is higher at the short frequency (Band 1) than at the other frequencies. We find that the spillover effect to agricultural commodities at Band 1 is 0.95, but at Bands 2 and 3, though it reduces, the effect varies in the respective assets – (higher for Coffee than Cotton); for energy, it reduces at Bands 2 and 3 as well, but highest at Band 1; the metals also experience a similar decreasing spillover effect; the stock markets however record the highest (FTSE, 2.13) and lowest (Nikkei, 0.09) spillover effect from CBDCAI in the network. CBDCAI records the least ABS from other markets at 0.54 – indicating that the assets do not highly correlate with CBDCAI and has little causality (WTH) to the assets at 0.71 in the short-term. This arguably is attributable to the fact that CBDCs are centralised and controlled financial assets which influences the level of risk in the price volatilities and uncertainties. Because of the likelihood of controlled risk effect [84], showed that CBDCs provide hedging effects to other assets. This is in line with our results which reiterate the fact that there is less correlation and little causality with other assets making it a better option to prevent systemic risk [55]. In Band 2 however, CBDCAI has the highest ABS index depicting the level of correlation to the assets as opposed to 0.02 in Band 3 irrespective of the decreasing causality. Thus, we observe that CBDCAI and assets are more interdependent in the range of month to semi-annual (Band 2) as compared to the other band ranges and has more causality effect even though relatively low, but in Band 1. When investors realise the hedging benefits that CBDCs has in a portfolio, they may adapt and rebalance their portfolios to using as hedging instruments against risk in the short-term. This hedging effect, however, dwindles away in the medium-to long-term because investors start to move to using CBDCs to diversify against risk. Implicitly, our findings are in line with [55,74] who showed that financial markets are less sensitive to CBDCAI.

The pairwise net spillovers in Table 4 are pair-specific and frequency-dependent [83]. At higher frequencies, the pairwise net spillover is high but gradually reduces across the bands for each pair. We also observe that pairs of CBDCAI and other assets over the bands averagely decrease.

**Table 4:** Pairwise net directional spillover between assets and CBDCAI.

Band 1: 3.14 to 0.79; corresponds to 1–4 Weeks												
Coffee-Cotton	Coffee-Crude Oil	Coffee-Natural Gas	Coffee-Gold	Coffee-Palladium	Coffee-Platinum	Coffee-Silver	Coffee-DJI	Coffee-FTSE	Coffee-Nikkei	Coffee-SP500	Coffee-CBDCAI	Cotton-Crude Oil
0.1080	−0.0111	−0.0251	0.0242	0.1287	0.1463	0.1480	0.0612	0.0063	−0.0076	0.0585	−0.0386	0.0450
Cotton-Natural Gas	Cotton-Gold	Cotton-Palladium	Cotton-Platinum	Cotton-Silver	Cotton-DJI	Cotton-FTSE	Cotton-Nikkei	Cotton-SP500	Cotton-CBDCAI	Crude Oil-Natural Gas	Crude Oil-Gold	Crude Oil-Palladium
−0.0356	0.0033	−0.0072	0.0630	0.0210	0.1966	0.1223	0.0946	0.2052	−0.0554	0.0205	0.0134	0.0497
Crude Oil-Platinum	Crude Oil-Silver	Crude Oil-DJI	Crude Oil-FTSE	Crude Oil-Nikkei	Crude Oil-SP500	Crude Oil-CBDCAI	Natural Gas-Gold	Natural Gas-Palladium	Natural Gas-Platinum	Natural Gas-Silver	Natural Gas-DJI	Natural Gas-FTSE
0.1363	0.0722	0.1734	0.1356	0.0811	0.1591	−0.0259	0.0121	−0.0012	−0.0505	0.0006	−0.0201	−0.0411
Natural Gas-Nikkei	Natural Gas-SP500	Natural Gas-CBDCAI	Gold–Palladium	Gold–Platinum	Gold–Silver	Gold-DJI	Gold-FTSE	Gold-Nikkei	Gold-SP500	Gold-CBDCAI	Palladium–Platinum	Palladium–Silver
−0.0305	−0.0164	−0.0485	−0.0316	0.2030	0.3227	−0.0086	0.0222	−0.0131	−0.0035	−0.0120	0.1821	0.1904
Palladium-DJI	Palladium-FTSE	Palladium-Nikkei	Palladium-SP500	Palladium-CBDCAI	Platinum–Silver	Platinum-DJI	Platinum-FTSE	Platinum-Nikkei	Platinum-SP500	Platinum-CBDCAI	Silver-DJI	Silver-FTSE
0.1026	0.0429	−0.0013	0.0724	−0.0047	−0.0099	0.0746	0.0436	−0.0402	0.0512	−0.0274	0.0619	0.0257
Silver-Nikkei	Silver-SP500	Silver-CBDCAI	DJI-FTSE	DJI-Nikkei	DJI-SP500	DJI-CBDCAI	FTSE-Nikkei	FTSE-SP500	FTSE-CBDCAI	Nikkei-SP500	Nikkei-CBDCAI	SP500-CBDCAI
−0.0218	0.0537	−0.0061	−0.2836	−0.2884	−0.0645	−0.0099	−0.0359	0.2265	−0.1432	0.2343	−0.0015	−0.0052
*Band 2: 0.79 to 0.13; corresponds to 4 to 24 Weeks*												
Coffee-Cotton	Coffee-Crude Oil	Coffee-Natural Gas	Coffee-Gold	Coffee-Palladium	Coffee-Platinum	Coffee-Silver	Coffee-DJI	Coffee-FTSE	Coffee-Nikkei	Coffee-SP500	Coffee-CBDCAI	Cotton-Crude Oil
−0.0083	0.0121	0.0092	−0.0472	0.0127	−0.0116	−0.0235	0.0017	−0.0007	−0.0094	0.0011	−0.0041	0.0803
Cotton-Natural Gas	Cotton-Gold	Cotton-Palladium	Cotton-Platinum	Cotton-Silver	Cotton-DJI	Cotton-FTSE	Cotton-Nikkei	Cotton-SP500	Cotton-CBDCAI	Crude Oil-Natural Gas	Crude Oil-Gold	Crude Oil-Palladium
−0.0266	−0.0108	0.0049	0.0190	0.0174	0.1259	0.1181	0.0594	0.1368	−0.0035	−0.0175	0.0040	0.0670
Crude Oil-Platinum	Crude Oil-Silver	Crude Oil-DJI	Crude Oil-FTSE	Crude Oil-Nikkei	Crude Oil-SP500	Crude Oil-CBDCAI	Natural Gas-Gold	Natural Gas-Palladium	Natural Gas-Platinum	Natural Gas-Silver	Natural Gas-DJI	Natural Gas-FTSE
0.0757	0.0084	0.0542	0.1340	0.0739	0.0604	0.0033	0.0154	−0.0081	0.0016	−0.0004	0.0287	−0.0027
Natural Gas-Nikkei	Natural Gas-SP500	Natural Gas-CBDCAI	Gold–Palladium	Gold–Platinum	Gold–Silver	Gold-DJI	Gold-FTSE	Gold-Nikkei	Gold-SP500	Gold-CBDCAI	Palladium–Platinum	Palladium–Silver
0.0258	0.0376	−0.0108	0.0047	−0.0159	0.0368	−0.0016	0.0008	−0.0127	−0.0018	−0.0032	0.0182	0.0079
Palladium-DJI	Palladium-FTSE	Palladium-Nikkei	Palladium-SP500	Palladium-CBDCAI	Platinum–Silver	Platinum-DJI	Platinum-FTSE	Platinum-Nikkei	Platinum-SP500	Platinum-CBDCAI	Silver-DJI	Silver-FTSE
−0.0103	0.0393	0.0195	−0.0055	−0.0148	0.0128	0.0159	0.0886	0.0325	0.0182	−0.0022	−0.0044	0.0322
Silver-Nikkei	Silver-SP500	Silver-CBDCAI	DJI-FTSE	DJI-Nikkei	DJI-SP500	DJI-CBDCAI	FTSE-Nikkei	FTSE-SP500	FTSE-CBDCAI	Nikkei-SP500	Nikkei-CBDCAI	SP500-CBDCAI
0.0073	−0.0008	−0.0065	0.0599	−0.0527	−0.0005	−0.0005	−0.1344	−0.0444	−0.0001	0.0679	−0.0002	−0.0016
*Band 3: 0.13 to 0.00; corresponds to infinite weeks*												
Coffee-Cotton	Coffee-Crude Oil	Coffee-Natural Gas	Coffee-Gold	Coffee-Palladium	Coffee-Platinum	Coffee-Silver	Coffee-DJI	Coffee-FTSE	Coffee-Nikkei	Coffee-SP500	Coffee-CBDCAI	Cotton-Crude Oil
−0.0020	0.0035	0.0028	−0.0124	0.0029	−0.0031	−0.0063	0.0003	−0.0002	−0.0026	0.0002	−0.0009	0.0217
Cotton-Natural Gas	Cotton-Gold	Cotton-Palladium	Cotton-Platinum	Cotton-Silver	Cotton-DJI	Cotton-FTSE	Cotton-Nikkei	Cotton-SP500	Cotton-CBDCAI Cru	de_Oil-Natural Gas	Crude Oil-Gold	Crude Oil-Palladium
−0.0076	−0.0028	0.0012	0.0052	0.0046	0.0335	0.0320	0.0157	0.0366	−0.0008	−0.0052	0.0010	0.0175
Crude Oil-Platinum	Crude Oil-Silver	Crude Oil-DJI	Crude Oil-FTSE	Crude Oil-Nikkei	Crude Oil-SP500	Crude Oil-CBDCAI	Natural Gas-Gold	Natural Gas-Palladium	Natural Gas-Platinum	Natural Gas-Silver	Natural Gas-DJI	Natural Gas-FTSE
0.0194	0.0017	0.0147	0.0368	0.0196	0.0165	0.0007	0.0042	−0.0021	0.0005	−0.0001	0.0079	−0.0006
Natural Gas-Nikkei	Natural Gas-SP500	Natural Gas-CBDCAI	Gold–Palladium	Gold–Platinum	Gold–Silver	Gold-DJI	Gold-FTSE	Gold-Nikkei	Gold-SP500	Gold-CBDCAI	Palladium–Platinum	Palladium–Silver
0.0070	0.0103	−0.0027	0.0010	−0.0047	0.0085	−0.0005	0.0001	−0.0029	−0.0006	−0.0008	0.0048	0.0018
Palladium-DJI	Palladium-FTSE	Palladium-Nikkei	Palladium-SP500	Palladium-CBDCAI	Platinum–Silver	Platinum-DJI	Platinum-FTSE	Platinum-Nikkei	Platinum-SP500	Platinum-CBDCAI	Silver-DJI	Silver-FTSE
−0.0029	0.0096	0.0049	−0.0016	−0.0038	0.0031	0.0042	0.0230	0.0084	0.0050	−0.0006	−0.0011	0.0083
Silver-Nikkei	Silver-SP500	Silver-CBDCAI	DJI-FTSE	DJI-Nikkei	DJI-SP500	DJI-CBDCAI	FTSE-Nikkei	FTSE-SP500	FTSE-CBDCAI	Nikkei-SP500	Nikkei-CBDCAI	SP500-CBDCAI
0.0020	−0.0002	−0.0016	0.0154	−0.0144	0.0000	−0.0001	−0.0353	−0.0112	0.0002	0.0187	0.0000	−0.0003

Note: All values are in percentages. The pairwise spillover indexes show an asset's net contribution to the volatility of another asset [85].

The article "Connectedness in cross-assets and digital assets attention indices" was published in 2023. Journal: Heliyon.

The rolling spillover for the assets and CBDCAI are in Fig. 4 (overall) and Fig. 5 (pairwise net). In Fig. 4, we observe a 62.5 % connectedness at band 1 in early 2016 which plunges and reduces to 57.5 % in late 2016. In bands 2 and 3, the fluctuations in the graphs are similar with a spike in 2016. The pairwise net spillover plots confirm the outputs in Table 4 where the graphs are unique to the pair and vary uniquely at respective frequencies.

**Fig. 4:** Overall rolling spillover between 12 cross-assets and CBDCAI. Note: Band 1 is the short-term frequency (monthly); Band 2 is the medium-term frequency (month-semi annual); Band 3 is the long-term frequency (semi-annual to infinity).

**Fig. 5:** Pairwise net rolling spillover between 12 cross-assets and CBDCAI. Note: The pairwise spillover indexes show an asset's net contribution to the volatility of another asset [85]. The pairwise net directional connectedness is pair-specific and frequency-dependent. The pairwise net directional connectedness magnitudes vary across frequencies. Panel A is the short-term frequency (monthly); Panel B is the medium-term frequency (month-semi annual); Panel C is the long-term frequency (semi-annual to infinity).

Table 6, Table 7 and Fig. 6, Fig. 7 present the static and rolling spillovers of the assets and ICEA. The spillover indices in the table are invariably highest at a high frequency (Band 1) [58,71]. The spillover indices are high at 37.30, and reduces to 8.04 and 2.03 at bands 2 and 3 respectively. As well, we explore the spillover effect from ICEA to the assets and the indices show that over the frequency, this spillover effect reduces. The connectedness from ICEA to the assets is more dominant for Silver at bands 1 (1.11), 2(0.41) and Coffee (0.22), DJI at bands 1 (0.83) and 3 (0.27). In Table 5, the pairwise net spillover also show a pair -specific and frequency-dependent variations but higher in band 1 than in bands 2 and 3. Averagely, we observe that interdependently, all the variables take turns at respective bands and are either net transmitters or receivers. At band 1, Platinum, Silver, DJI, SP500 and ICEA are net transmitters; at band 2, Cotton, Crude oil, Natural gas, Gold, Palladium, Platinum, Nikkei and ICEA are net receivers and at band 3, Coffee, Gold, Palladium, Silver, DJI, FTSE and SP500 are net transmitters. Dominantly, ICEA interchangeably transmits and receives shock from the other assets at different horizons. Investors are sentimental. Thus, how they feel about cryptocurrency, and the level of mining and usage influence its volatility. This explains why it does not have a dominance but at different horizons, is a transmitter (short- and long-term) or a receiver (medium-term). Here, we report that the spillover effect from ICEA to Crude oil is a transmitter effect across bands, it is not as strong as what [74] may have reported. Across the bands, however, these net transmitter and net receiver indices are persistently decreasing [58,71].

**Table 5:** Total and net spillover indices between the assets and ICEA.

	Coffee	Cotton	Crude Oil	Natural Gas	Gold	Palladium	Platinum	Silver	DJI	FTSE	Nikkei	SP500	ICEA	FROM_ABS^a^	FROM_WTH^b^
*Band 1: 3.14 to 0.79; corresponds to 1 to 4 Weeks*															
Coffee	69.94	1.55	0.56	0.62	1.95	1.82	2.23	2.47	0.40	0.39	0.04	0.42	1.30	1.06	1.32
Cotton	0.40	53.83	1.76	1.39	0.40	0.51	1.78	0.49	4.88	2.91	1.48	4.95	0.41	1.64	2.06
Crude Oil	0.59	1.19	39.04	1.15	0.33	2.64	4.02	2.76	4.90	5.58	2.22	4.68	0.17	2.33	2.91
Natural Gas	0.98	1.69	1.14	72.73	0.48	0.50	0.07	0.04	1.16	0.08	0.51	1.34	1.97	0.77	0.96
Gold	2.13	0.15	0.13	0.3	36.18	7.17	11.6	22.53	0.06	0.38	0.80	0.08	0.24	3.50	4.39
Palladium	0.18	0.58	2.05	0.53	7.26	38.13	11.93	10.22	3.56	3.06	1.95	2.66	0.21	3.40	4.26
Platinum	0.49	0.99	2.31	0.74	9.24	9.69	30.61	12.79	3.55	3.57	1.29	2.95	0.17	3.68	4.60
Silver	0.89	0.18	1.98	0.06	18.84	8.14	13.06	30.46	2.19	1.37	0.21	2.07	0.55	3.81	4.77
DJI	0.09	2.41	2.69	1.44	0.27	2.17	2.64	1.56	23.31	11.70	10.53	21.71	0.24	4.42	5.53
FTSE	0.42	1.44	3.75	0.31	0.04	2.39	2.78	0.91	15.39	27.11	11.88	14.28	0.08	4.13	5.17
Nikkei	0.51	0.64	1.44	0.62	0.91	1.82	1.71	0.41	14.02	12.32	30.59	13.62	0.1	3.70	4.64
SP500	0.10	2.37	2.66	1.59	0.26	1.67	2.31	1.55	22.63	11.33	10.81	24.00	0.31	**4.43**	**5.55**
ICEA	0.54	0.24	0.33	0.01	0.42	0.43	0.31	1.11	0.83	0.21	0.59	0.69	77.14	0.44	0.55
TO_ABS^a^	0.56	1.03	1.60	0.67	3.11	3.00	4.19	4.37	5.66	4.07	3.26	5.34	0.44	***37.30***	
TO_WTH^b^	0.71	1.29	2.00	0.84	3.89	3.75	5.24	5.48	7.09	5.10	4.08	6.69	0.55		***46.72***
Net	−0.49	−0.61	−0.73	−0.09	−0.40	−0.40	0.51	0.56	1.24	−0.06	−0.45	0.91	0.00		
*Band 2: 0.79 to 0.13; corresponds to 4 to 24 Weeks*															
Coffee	12.29	0.02	0.27	0.21	0.04	0.15	0.01	0.04	0.04	0.00	0.01	0.03	0.01	0.06	0.40
Cotton	0.11	11.54	1.15	0.52	0.00	0.10	0.48	0.20	1.53	1.41	0.71	1.77	0.18	0.63	3.90
Crude Oil	0.02	0.19	12.26	0.04	0.13	1.22	2.05	1.10	1.58	2.82	1.24	1.59	0.09	**0.93**	**5.76**
Natural Gas	0.04	0.65	0.34	11.55	0.27	0.01	0.02	0.02	0.22	0.00	0.24	0.32	0.19	0.18	1.11
Gold	0.74	0.11	0.06	0.02	6.85	1.00	1.73	3.94	0.01	0.01	0.17	0.01	0.02	0.60	3.74
Palladium	0.04	0.01	0.31	0.12	1.15	6.99	1.97	1.55	0.47	0.80	0.36	0.35	0.08	0.56	3.45
Platinum	0.19	0.33	0.99	0.02	2.04	1.70	5.65	2.82	0.78	1.54	0.46	0.72	0.02	0.89	5.54
Silver	0.30	0.01	0.91	0.01	3.54	1.36	2.54	5.88	0.36	0.55	0.08	0.40	0.04	0.78	4.83
DJI	0.01	0.27	0.85	0.01	0.03	0.60	0.59	0.45	3.77	3.27	1.94	3.60	0.01	0.89	5.56
FTSE	0.02	0.28	1.14	0.04	0.00	0.33	0.42	0.22	2.58	5.85	1.88	2.58	0.01	0.73	4.54
Nikkei	0.19	0.27	0.49	0.00	0.37	0.18	0.10	0.01	2.85	3.64	5.86	3.03	0.01	0.86	5.31
SP500	0.01	0.33	0.74	0.01	0.03	0.41	0.50	0.44	3.52	3.01	1.88	3.85	0.02	0.84	5.20
ICEA	0.22	0.02	0.07	0.00	0.14	0.13	0.08	0.41	0.06	0.00	0.00	0.05	12.56	0.09	0.57
TO_ABS^a^	0.14	0.19	0.56	0.08	0.60	0.55	0.81	0.86	1.08	1.31	0.69	1.11	0.05	***8.04***	
TO_WTH^b^	0.90	1.19	3.50	0.47	3.70	3.43	5.01	5.34	6.68	8.15	4.28	6.90	0.33		***49.90***
Net	0.08	−0.44	−0.36	−0.10	−0.01	−0.00	−0.09	0.08	0.18	0.58	−0.17	0.27	−0.04		
*Band 3: 0.13 to 0.00; corresponds to infinite weeks*															
Coffee	3.01	0.00	0.07	0.05	0.00	0.03	0.00	0.00	0.01	0.00	0.00	0.01	0.00	0.01	0.35
Cotton	0.03	2.93	0.31	0.13	0.00	0.02	0.13	0.05	0.40	0.38	0.19	0.46	0.05	0.17	4.09
Crude Oil	0.00	0.05	3.19	0.00	0.04	0.31	0.54	0.29	0.42	0.76	0.33	0.43	0.03	**0.25**	**6.09**
Natural Gas	0.00	0.17	0.09	2.85	0.07	0.00	0.00	0.00	0.06	0.00	0.06	0.09	0.05	0.05	1.14
Gold	0.19	0.03	0.02	0.00	1.68	0.24	0.42	0.96	0.00	0.00	0.04	0.00	0.01	0.15	3.61
Palladium	0.01	0.00	0.07	0.03	0.28	1.72	0.48	0.38	0.11	0.20	0.09	0.08	0.02	0.13	3.32
Platinum	0.05	0.09	0.27	0.00	0.51	0.41	1.41	0.71	0.2	0.40	0.12	0.19	0.00	0.23	5.59
Silver	0.07	0.00	0.24	0.00	0.87	0.33	0.64	1.47	0.09	0.15	0.02	0.10	0.01	0.20	4.82
DJI	0.00	0.07	0.22	0.00	0.01	0.15	0.15	0.12	0.93	0.83	0.48	0.9	0.00	0.22	5.54
FTSE	0.00	0.07	0.30	0.01	0.00	0.08	0.11	0.06	0.65	1.47	0.47	0.65	0.00	0.18	4.57
Nikkei	0.05	0.07	0.13	0.00	0.09	0.04	0.03	0.00	0.72	0.93	1.46	0.77	0.00	0.22	5.38
SP500	0.00	0.08	0.19	0.00	0.01	0.10	0.13	0.11	0.87	0.76	0.46	0.95	0.00	0.21	5.17
ICEA	0.05	0.01	0.02	0.00	0.04	0.03	0.02	0.10	0.01	0.00	0.00	0.01	3.10	0.02	0.56
TO_ABS^a^	0.04	0.05	0.15	0.02	0.15	0.14	0.20	0.21	0.27	0.34	0.17	0.28	0.01	***2.03***	
TO_WTH^b^	0.87	1.24	3.66	0.45	3.63	3.35	5.03	5.30	6.72	8.34	4.30	7.01	0.33		***50.24***
Net	0.02	−0.12	−0.10	−0.03	0.00	0.00	−0.02	0.02	0.05	0.15	−0.04	0.08	−0.009		

Note.

a Absolute to measures return spillovers from asset m to other assets. Absolute from measures return spillovers from other assets to asset m.

b Within to measures return spillovers from asset m to other assets, including from own innovations to asset n. Within from measures return spillovers from other assets to asset m, including from own innovations to asset n [71,83]. The largest contributions of assets per frequency band are in bold italics. Positive **Net** denotes that the asset is a **net transmitter** [an asset that can dominate and cause systemic risk; lead the price fluctuations in other assets] while negative **Net** denote **net recipient** [an asset that is less dominant and more vulnerable to external shocks].

The article "Connectedness in cross-assets and digital assets attention indices" was published in 2023. Journal: Heliyon.

**Table 6:** Pairwise net directional spillover between assets and ICEA.

Band 1: 3.14 to 0.79; corresponds to 1–4 Weeks												
Coffee-Cotton	Coffee-Crude Oil	Coffee-Natural Gas	Coffee-Gold	Coffee-Palladium	Coffee-Platinum	Coffee-Silver	Coffee-DJI	Coffee-FTSE	Coffee-Nikkei	Coffee-SP500	Coffee-ICEA	Cotton-Crude Oil
0.0880	−0.0028	−0.0279	−0.0136	0.1256	0.1337	0.1217	0.0239	−0.0020	−0.0363	0.0248	0.0579	0.0438
Cotton-Natural Gas	Cotton-Gold	Cotton-Palladium	Cotton-Platinum	Cotton-Silver	Cotton-DJI	Cotton-FTSE	Cotton-Nikkei	Cotton-SP500	Cotton-ICEA	Crude_Oil-Natural Gas	Crude Oil-Gold	Crude Oil-Palladium
−0.0234	0.0196	−0.0055	0.0608	0.0238	0.1898	0.1132	0.0648	0.1983	0.0131	0.0013	0.0150	0.0454
Crude Oil-Platinum	Crude Oil-Silver	Crude Oil-DJI	Crude Oil-FTSE	Crude Oil-Nikkei	Crude Oil-SP500	Crude Oil-ICEA	Natural Gas-Gold	Natural Gas-Palladium	Natural Gas-Platinum	Natural Gas-Silver	Natural Gas-DJI	Natural Gas-FTSE
0.1318	0.0601	0.1700	0.1409	0.0606	0.1554	−0.0118	0.0139	−0.0022	−0.0520	−0.0014	−0.0214	−0.0174
Natural Gas-Nikkei	Natural Gas-SP500	Natural Gas-ICEA	Gold–Palladium	Gold–Platinum	Gold–Silver	Gold-DJI	Gold-FTSE	Gold-Nikkei	Gold-SP500	Gold-ICEA	Palladium–Platinum	Palladium–Silver
−0.0088	−0.0196	0.1508	−0.0071	0.1820	0.2838	−0.0158	0.0260	−0.0086	−0.0141	−0.0138	0.1724	0.1600
Palladium-DJI	Palladium-FTSE	Palladium-Nikkei	Palladium-SP500	Palladium-ICEA	Platinum–Silver	Platinum-DJI	Platinum-FTSE	Platinum-Nikkei	Platinum-SP500	Platinum-ICEA	Silver-DJI	Silver-FTSE
0.1070	0.0510	0.0094	0.0755	−0.0170	−0.0213	0.0704	0.0606	−0.0318	0.0491	−0.0102	0.0482	0.0358
Silver-Nikkei	Silver-SP500	Silver-ICEA	DJI-FTSE	DJI-Nikkei	DJI-SP500	DJI-ICEA	FTSE-Nikkei	FTSE-SP500	FTSE-ICEA	Nikkei-SP500	Nikkei-ICEA	SP500-ICEA
−0.0154	0.0399	−0.0428	−0.2844	−0.2687	−0.0710	−0.0447	−0.0341	0.2273	−0.0100	0.2165	−0.0373	−0.0298
*Band 2: 0.79 to 0.13; corresponds to 4 to 24 Weeks*												
Coffee-Cotton	Coffee-Crude Oil	Coffee-Natural Gas	Coffee-Gold	Coffee-Palladium	Coffee-Platinum	Coffee-Silver	Coffee-DJI	Coffee-FTSE	Coffee-Nikkei	Coffee-SP500	Coffee-ICEA	Cotton-Crude Oil
−0.0067	0.0196	0.0131	−0.0539	0.0084	−0.0135	−0.0201	0.0017	−0.0015	−0.0134	0.0020	−0.0162	0.0738
Cotton-Natural Gas	Cotton-Gold	Cotton-Palladium	Cotton-Platinum	Cotton-Silver	Cotton-DJI	Cotton-FTSE	Cotton-Nikkei	Cotton-SP500	Cotton-ICEA	Crude Oil-Natural Gas	Crude Oil-Gold	Crude Oil-Palladium
−0.0098	−0.0084	0.0062	0.0118	0.0145	0.0971	0.0873	0.0338	0.1112	0.0125	−0.0235	0.0056	0.0700
Crude Oil-Platinum	Crude Oil-Silver	Crude Oil-DJI	Crude Oil-FTSE	Crude Oil-Nikkei	Crude Oil-SP500	Crude Oil-ICEA	Natural Gas-Gold	Natural Gas-Palladium	Natural Gas-Platinum	Natural Gas-Silver	Natural Gas-DJI	Natural Gas-FTSE
0.0816	0.0143	0.0562	0.1288	0.0574	0.0657	0.0018	0.0195	−0.0086	0.0000	0.0006	0.0160	−0.0026
Natural Gas-Nikkei	Natural Gas-SP500	Natural Gas-ICEA	Gold–Palladium	Gold–Platinum	Gold–Silver	Gold-DJI	Gold-FTSE	Gold-Nikkei	Gold-SP500	Gold-ICEA	Palladium–Platinum	Palladium–Silver
0.0178	0.0242	0.0148	−0.0110	−0.0244	0.0311	−0.0013	0.0003	−0.0153	−0.0018	−0.0090	0.0206	0.0151
Palladium-DJI	Palladium-FTSE	Palladium-Nikkei	Palladium-SP500	Palladium-ICEA	Platinum–Silver	Platinum-DJI	Platinum-FTSE	Platinum-Nikkei	Platinum-SP500	Platinum-ICEA	Silver-DJI	Silver-FTSE
−0.0100	0.0365	0.0143	−0.0049	−0.0038	0.0212	0.0148	0.0859	0.0278	0.0171	−0.0048	−0.0067	0.0258
Silver-Nikkei	Silver-SP500	Silver-ICEA	DJI-FTSE	DJI-Nikkei	DJI-SP500	DJI-ICEA	FTSE-Nikkei	FTSE-SP500	FTSE-ICEA	Nikkei-SP500	Nikkei-ICEA	SP500-ICEA
0.0061	−0.0034	−0.0284	0.0535	−0.0697	0.0067	−0.0037	−0.1357	−0.0328	0.0006	0.0882	0.0008	−0.0023
*Band 3: 0.13 to 0.00; corresponds to infinite weeks*												
Coffee-Cotton	Coffee-Crude Oil	Coffee-Natural Gas	Coffee-Gold	Coffee-Palladium	Coffee-Platinum	Coffee-Silver	Coffee-DJI	Coffee-FTSE	Coffee-Nikkei	Coffee-SP500	Coffee-ICEA	Cotton-Crude Oil
−0.0017	0.0054	0.0036	−0.0140	0.0018	−0.0035	−0.0053	0.0004	−0.0003	−0.0034	0.0004	−0.0042	0.0199
Cotton-Natural Gas	Cotton-Gold	Cotton-Palladium	Cotton-Platinum	Cotton-Silver	Cotton-DJI	Cotton-FTSE	Cotton-Nikkei	Cotton-SP500	Cotton-ICEA	Crude Oil-Natural Gas	Crude Oil-Gold	Crude Oil-Palladium
−0.0031	−0.0023	0.0017	0.0033	0.0038	0.0254	0.0234	0.0089	0.0294	0.0032	−0.0066	0.0015	0.0186
Crude Oil-Platinum	Crude Oil-Silver	Crude Oil-DJI	Crude Oil-FTSE	Crude Oil-Nikkei	Crude Oil-SP500	Crude Oil-ICEA	Natural Gas-Gold	Natural Gas-Palladium	Natural Gas-Platinum	Natural Gas-Silver	Natural Gas-DJI	Natural Gas-FTSE
0.0212	0.0037	0.0155	0.0356	0.0155	0.0182	0.0006	0.0052	−0.0022	0.0001	0.0002	0.0043	−0.0007
Natural Gas-Nikkei	Natural Gas-SP500	Natural Gas-ICEA	Gold–Palladium	Gold–Platinum	Gold–Silver	Gold-DJI	Gold-FTSE	Gold-Nikkei	Gold-SP500	Gold-ICEA	Palladium–Platinum	Palladium–Silver
0.0047	0.0066	0.0036	−0.0033	−0.0070	0.0068	−0.0004	0.0001	−0.0036	−0.0005	−0.0023	0.0053	0.0036
Palladium-DJI	Palladium-FTSE	Palladium-Nikkei	Palladium-SP500	Palladium-ICEA	Platinum–Silver	Platinum-DJI	Platinum-FTSE	Platinum-Nikkei	Platinum-SP500	Platinum-ICEA	Silver-DJI	Silver-FTSE
−0.0029	0.0088	0.0034	−0.0015	−0.0009	0.0053	0.0039	0.0222	0.0072	0.0047	−0.0012	−0.0018	0.0066
Silver-Nikkei	Silver-SP500	Silver-ICEA	DJI-FTSE	DJI-Nikkei	DJI-SP500	DJI-ICEA	FTSE-Nikkei	FTSE-SP500	FTSE-ICEA	Nikkei-SP500	Nikkei-ICEA	SP500-ICEA
0.0016	−0.0008	−0.0072	0.0139	−0.0185	0.0020	−0.0009	−0.0354	−0.0082	0.0002	0.0237	0.0003	−0.0005

Note: All values are in percentages. The pairwise spillover indexes show an asset's net contribution to the volatility of another asset [85].

The article "Connectedness in cross-assets and digital assets attention indices" was published in 2023. Journal: Heliyon.

**Table 7:** Total and net spillover indices between the assets and NFTAI.

	Coffee	Cotton	Crude Oil	Natural Gas	Gold	Palladium	Platinum	Silver	DJI	FTSE	Nikkei	SP500	NFTAI	FROM_ABS^a^	FROM_WTH^b^
*Band 1: 3.14 to 0.79; corresponds to 1 to 4 Weeks*															
Coffee	66.59	0.96	0.22	1.38	3.03	2.14	1.30	2.27	0.94	0.92	0.36	0.97	0.49	1.15	1.44
Cotton	0.60	46.91	2.68	2.98	0.75	0.37	1.64	0.28	5.95	3.45	1.65	5.64	0.03	2.00	2.50
Crude Oil	0.22	1.56	34.10	0.78	0.57	2.99	5.69	4.71	4.44	4.45	3.42	4.09	0.62	2.58	3.22
Natural Gas	2.04	3.77	1.15	67.25	0.69	0.31	0.41	0.06	3.12	0.02	1.49	3.25	0.06	1.26	1.57
Gold	1.06	0.81	0.40	0.30	37.61	8.76	9.81	23.09	0.31	0.91	0.12	0.41	0.11	3.55	4.42
Palladium	0.70	0.65	2.01	0.52	9.71	37.81	11.56	10.27	2.98	3.16	2.78	1.98	0.23	3.58	4.47
Platinum	0.34	1.09	3.08	1.09	7.94	9.49	29.42	11.70	4.45	4.05	2.43	3.67	0.16	3.81	4.75
Silver	0.58	0.38	3.56	0.02	18.2	7.37	11.17	28.75	2.94	2.06	0.91	2.95	0.03	3.86	4.82
DJI	0.06	3.12	2.48	2.37	0.62	2.04	3.24	2.19	21.36	11.18	10.69	19.87	0.11	**4.46**	**5.56**
FTSE	0.16	2.07	2.85	0.72	0.54	2.59	3.30	1.58	14.39	24.85	11.8	12.48	0.00	4.04	5.04
Nikkei	0.13	0.90	1.72	1.62	0.41	2.70	3.18	1.35	14.62	12.28	27.17	13.79	0.03	4.06	5.06
SP500	0.09	2.99	2.43	2.52	0.61	1.48	2.90	2.34	21.08	10.31	10.86	22.34	0.18	4.44	5.55
NFTAI	0.19	0.51	0.91	2.66	0.36	1.34	0.18	0.16	0.14	0.17	0.14	0.19	86.58	0.53	0.67
TO_ABS^a^	0.47	1.45	1.81	1.30	3.34	3.20	4.18	4.62	5.80	4.07	3.59	5.33	0.16	***39.31***	
TO_WTH^b^	0.59	1.80	2.25	1.63	4.17	3.99	5.22	5.76	7.23	5.08	4.48	6.65	0.20		***49.06***
Net	−0.68	−0.56	−0.77	0.05	−0.21	−0.38	0.38	0.76	1.34	0.04	−0.47	0.89	−0.38		
*Band 2: 0.79 to 0.13; corresponds to 4 to 24 Weeks*															
Coffee	13.27	0.03	0.17	0.37	0.03	0.68	0.04	0.02	0.05	0.05	0.05	0.05	0.00	0.12	0.75
Cotton	0.03	10.5	1.90	0.80	0.00	0.02	0.75	0.16	1.98	1.94	1.15	2.13	0.01	0.84	5.29
Crude Oil	0.02	0.40	11.51	0.03	0.05	1.05	2.71	1.43	1.71	2.74	2.16	1.65	0.03	**1.07**	**6.8**
Natural Gas	0.10	1.04	0.08	10.5	0.09	0.00	0.04	0.00	0.34	0.00	0.48	0.43	0.00	0.20	1.27
Gold	0.46	0.33|	0.10	0.13	5.94	1.36	1.23	3.45	0.02	0.09	0.00	0.03	0.00	0.55	3.50
Palladium	0.00	0.00	0.31	0.06	1.02	6.19	1.95	1.11	0.36	0.81	0.47	0.23	0.08	0.49	3.11
Platinum	0.06	0.24	1.42	0.03	1.22	1.52	5.27	2.20	1.00	1.85	0.99	0.93	0.02	0.88	5.60
Silver	0.19	0.00	1.57	0.00	3.21	1.31	2.46	5.58	0.54	0.87	0.43	0.66	0.00	0.86	5.47
DJI	0.01	0.44	0.92	0.02	0.03	0.44	0.72	0.52	3.77	3.56	2.38	3.63	0.00	0.97	6.17
FTSE	0.03	0.50	1.31	0.06	0.05	0.23	0.57	0.27	2.96	6.35	2.74	2.85	0.00	0.89	5.64
Nikkei	0.12	0.34	0.66	0.01	0.13	0.17	0.27	0.08	2.64	3.56	5.24	2.73	0.00	0.82	5.22
SP500	0.01	0.50	0.80	0.02	0.05	0.26	0.60	0.57	3.59	3.19	2.28	3.94	0.00	0.91	5.78
NFTAI	0.01	0.04	0.06	0.11	0.00	0.01	0.01	0.00	0.00	0.00	0.05	0.00	4.94	0.02	0.14
TO_ABS^a^	0.08	0.30	0.72	0.13	0.45	0.54	0.87	0.75	1.17	1.44	1.01	1.18	0.01	***8.65***	
TO_WTH^b^	0.50	1.88	4.53	0.80	2.86	3.43	5.53	4.78	7.4	9.09	6.41	7.47	0.07		***54.74***
Net	−0.04	−0.54	−0.36	−0.07	−0.10	0.05	−0.01	−0.11	0.19	0.55	0.19	0.27	−0.01		
*Band 3: 0.13 to 0.00; corresponds to infinite weeks*															
Coffee	3.27	0.01	0.05	0.1	0.00	0.17	0.01	0.00	0.01	0.01	0.01	0.01	0.00	0.03	0.70
Cotton	0.00	2.71	0.53	0.2	0.00	0.01	0.21	0.05	0.54	0.54	0.32	0.59	0.00	0.23	5.66
Crude Oil	0.00	0.12	3.08	0.00	0.01	0.26	0.72	0.37	0.47	0.76	0.6	0.46	0.01	**0.29**	**7.19**
Natural Gas	0.02	0.27	0.02	2.61	0.02	0.00	0.01	0.00	0.09	0.00	0.12	0.11	0.00	0.05	1.26
Gold	0.12	0.08	0.02	0.03	1.43	0.32	0.29	0.83	0.00	0.02	0.00	0.01	0.00	0.13	3.28
Palladium	0.00	0.00	0.08	0.01	0.24	1.51	0.48	0.26	0.09	0.20	0.11	0.06	0.02	0.12	2.93
Platinum	0.01	0.07	0.39	0.01	0.29	0.37	1.34	0.56	0.27	0.50	0.27	0.25	0.01	0.23	5.66
Silver	0.04	0.00	0.42	0.00	0.77	0.31	0.63	1.40	0.14	0.23	0.12	0.18	0.00	0.22	5.41
DJI	0.00	0.12	0.25	0.00	0.01	0.11	0.19	0.14	0.96	0.92	0.61	0.93	0.00	0.25	6.22
FTSE	0.01	0.14	0.36	0.01	0.01	0.06	0.16	0.08	0.77	1.66	0.72	0.75	0.00	0.24	5.84
Nikkei	0.03	0.1	0.18	0.00	0.03	0.04	0.07	0.02	0.68	0.93	1.34	0.71	0.00	0.22	5.33
SP500	0.00	0.13	0.22	0.00	0.01	0.06	0.16	0.15	0.91	0.83	0.59	1.01	0.00	0.24	5.82
NFTAI	0.00	0.01	0.01	0.03	0.00	0.00	0.00	0.00	0.00	0.00	0.01	0.00	1.19	0.01	0.12
TO_ABS^a^	0.02	0.08	0.2	0.03	0.11	0.13	0.23	0.19	0.31	0.38	0.27	0.31	0.00	***2.25***	
TO_WTH^b^	0.44	1.99	4.83	0.75	2.62	3.23	5.57	4.65	7.55	9.39	6.63	7.7	0.07		***55.42***
Net	−0.01	−0.15	−0.10	−0.02	−0.03	0.01	0.00	−0.03	0.05	0.14	0.05	0.08	0.00		

Note.

a Absolute to measures return spillovers from asset m to other assets. Absolute from measures return spillovers from other assets to asset m.

b Within to measures return spillovers from asset m to other assets, including from own innovations to asset n. Within from measures return spillovers from other assets to asset m, including from own innovations to asset n [71,83]. The largest contributions of assets per frequency band are in bold italics. Positive **Net** denotes that the asset is a **net transmitter** [an asset that can dominate and cause systemic risk; lead the price fluctuations in other assets] while negative **Net** denote **net recipient** [an asset that is less dominant and more vulnerable to external shocks].

The article "Connectedness in cross-assets and digital assets attention indices" was published in 2023. Journal: Heliyon.

**Fig. 6:** Overall rolling spillover between 12 cross-assets and ICEA Note: Band 1 is the short-term frequency (monthly); Band 2 is the medium-term frequency (month-semi annual); Band 3 is the long-term frequency (semi-annual to infinity).

**Fig. 7:** Pairwise net rolling spillover between 12 cross-assets and ICEA Note: The pairwise spillover indexes show an asset's net contribution to the volatility of another asset [85]. The pairwise net directional connectedness is pair-specific and frequency-dependent. The pairwise net directional connectedness magnitudes vary across frequencies. Panel A is the short-term frequency (monthly); Panel B is the medium-term frequency (month-semi annual); Panel C is the long-term frequency (semi-annual to infinity).

The rolling spillover also shows a frequency varying spillover between the assets and ICEA. The overall spillover in Fig. 6 has varying fluctuations in respective bands. At band 1, there is an upsurge at 80 % in 2015, gradual fluctuations then a sharp hike downwards at 45 %. Band 2 has a more fluctuating and steady variation but band 3 shows a more persistent fluctuation but in 2018, plunges to 20 %. The pairwise net rolling spillover here also depicts a pair-specific and frequency-dependent spillover across the bands.

Table 7, Table 8, and Fig. 8, Fig. 9 show the static and rolling spillover for the assets and NFTAI. Fig. 8 shows a gradual progression in the fluctuations with plunges at 2017 at varying percentiles. Fig. 9 depict a varying pair-specific-frequency-dependent fluctuation across bands. From Table 7, the correlations between the variables decrease in bands 2 (8.65) and 3 (2.25) but is high at band 1 (39.31). The static net spillover effect between NFTAI and the assets show that averagely, Cotton, Coffee, Crude oil and Gold are net receivers across the bands, Silver at bands 2 and 3 and Palladium, Nikkei and NFTAI at band 1 and Platinum at band 2. Varyingly, these net spillovers reduce across bands. Unlike [50], who found that NFTs are volatility spillover receivers, our results show that it is only true at the short-term and mostly, NFTs are net return transmitters. This is reflective of investors increasing interest in NFTs which has caused speculative and increased price fluctuations. Thus, implicitly, our result imply that attention from NFTs move the prices of other cross-assets. NFTAI dominating net receiver property shows that independently, it has the ability to move other assets; theoretically, this caould be attributed to the fact that most NFTs are built on cryptocurrencies. The spillover effect from NFTAI to the assets is highest at band 1 and recorded by Natural gas (2.66), followed by Palladium (1.34) and the other assets, averaging between 0.19 and 0.51. At band 2, though the degree of effect is reducing, Crude oil has the highest spillover effect at 0.06 and Natural gas at 0.03 at band 3.

**Table 8:** Pairwise net directional spillover between assets and NFTAI.

Band 1: 3.14 to 0.79; corresponds to 1–4 Weeks												
Coffee-Cotton	Coffee-Crude Oil	Coffee-Natural Gas	Coffee-Gold	Coffee-Palladium	Coffee-Platinum	Coffee-Silver	Coffee-DJI	Coffee-FTSE	Coffee-Nikkei	Coffee-SP500	Coffee-NFTAI	Cotton-Crude Oil
0.0273	−0.0005	−0.0510	0.1516	0.1105	0.0737	0.1303	0.0674	0.0580	0.0178	0.0679	0.0234	0.0857
Cotton-Natural Gas	Cotton-Gold	Cotton-Palladium	Cotton-Platinum	Cotton-Silver	Cotton-DJI	Cotton-FTSE	Cotton-Nikkei	Cotton-SP500	Cotton-NFTAI	Crude Oil-Natural Gas	Crude Oil-Gold	Crude Oil-Palladium
−0.0608	−0.0043	−0.0218	0.0429	−0.0077	0.2176	0.1064	0.0577	0.2035	−0.0367	−0.0279	0.0131	0.0753
Crude Oil-Platinum	Crude Oil-Silver	Crude Oil-DJI	Crude Oil-FTSE	Crude Oil-Nikkei	Crude Oil-SP500	Crude Oil-NFTAI	Natural Gas-Gold	Natural Gas-Palladium	Natural Gas-Platinum	Natural Gas-Silver	Natural Gas-DJI	Natural Gas-FTSE
0.2008	0.0880	0.1506	0.1234	0.1309	0.1279	−0.0221	0.0296	−0.0160	−0.0522	0.0036	0.0576	−0.0539
Natural Gas-Nikkei	Natural Gas-SP500	Natural Gas-NFTAI	Gold–Palladium	Gold–Platinum	Gold–Silver	Gold-DJI	Gold-FTSE	Gold-Nikkei	Gold-SP500	Gold-NFTAI	Palladium–Platinum	Palladium–Silver
−0.0100	0.0563	−0.2003	−0.0729	0.1441	0.3764	−0.0239	0.0281	−0.0223	−0.0151	−0.0189	0.1596	0.2232
Palladium-DJI	Palladium-FTSE	Palladium-Nikkei	Palladium-SP500	Palladium-NFTAI	Platinum–Silver	Platinum-DJI	Platinum-FTSE	Platinum-Nikkei	Platinum-SP500	Platinum-NFTAI	Silver-DJI	Silver-FTSE
0.0724	0.0441	0.0063	0.0385	−0.0855	0.0410	0.0933	0.0577	−0.0574	0.0596	−0.0018	0.0580	0.0374
Silver-Nikkei	Silver-SP500	Silver-NFTAI	DJI-FTSE	DJI-Nikkei	DJI-SP500	DJI-NFTAI	FTSE-Nikkei	FTSE-SP500	FTSE-NFTAI	Nikkei-SP500	Nikkei-NFTAI	SP500-NFTAI
−0.0338	0.0470	−0.0101	−0.2465	−0.3026	−0.0930	−0.0026	−0.0372	0.1671	−0.0127	0.2251	−0.0084	−0.0007
*Band 2: 0.79 to 0.13; corresponds to 4 to 24 Weeks*												
Coffee-Cotton	Coffee-Crude Oil	Coffee-Natural Gas	Coffee-Gold	Coffee-Palladium	Coffee-Platinum	Coffee-Silver	Coffee-DJI	Coffee-FTSE	Coffee-Nikkei	Coffee-SP500	Coffee-NFTAI	Cotton-Crude Oil
0.0006	0.0112	0.0210	−0.0328	0.0520	−0.0015	−0.0128	0.0033	0.0016	−0.0056	0.0033	−0.0002	0.1153
Cotton-Natural Gas	Cotton-Gold	Cotton-Palladium	Cotton-Platinum	Cotton-Silver	Cotton-DJI	Cotton-FTSE	Cotton-Nikkei	Cotton-SP500	Cotton-NFTAI	Crude Oil-Natural Gas	Crude Oil-Gold	Crude Oil-Palladium
−0.0181	−0.0248	0.0017	0.0394	0.0124	0.1187	0.1103	0.0621	0.1257	−0.0027	−0.0041	−0.0040	0.0568
Crude Oil-Platinum	Crude Oil-Silver	Crude Oil-DJI	Crude Oil-FTSE	Crude Oil-Nikkei	Crude Oil-SP500	Crude Oil-NFTAI	Natural Gas-Gold	Natural Gas-Palladium	Natural Gas-Platinum	Natural Gas-Silver	Natural Gas-DJI	Natural Gas-FTSE
0.0991	−0.0113	0.0603	0.1097	0.1161	0.0655	−0.0023	−0.0033	−0.0042	0.0009	0.0000	0.0249	−0.0042
Natural Gas-Nikkei	Natural Gas-SP500	Natural Gas-NFTAI	Gold–Palladium	Gold–Platinum	Gold–Silver	Gold-DJI	Gold-FTSE	Gold-Nikkei	Gold-SP500	Gold-NFTAI	Palladium–Platinum	Palladium–Silver
0.0361	0.0316	−0.0082	0.0260	0.0006	0.0182	−0.0008	0.0033	−0.0095	−0.0010	0.0000	0.0328	−0.0150
Palladium-DJI	Palladium-FTSE	Palladium-Nikkei	Palladium-SP500	Palladium-NFTAI	Platinum–Silver	Platinum-DJI	Platinum-FTSE	Platinum-Nikkei	Platinum-SP500	Platinum-NFTAI	Silver-DJI	Silver-FTSE
−0.0062	0.0444	0.0230	−0.0023	0.0054	−0.0201	0.0217	0.0980	0.0555	0.0256	0.0012	0.0013	0.0462
Silver-Nikkei	Silver-SP500	Silver-NFTAI	DJI-FTSE	DJI-Nikkei	DJI-SP500	DJI-NFTAI	FTSE-Nikkei	FTSE-SP500	FTSE-NFTAI	Nikkei-SP500	Nikkei-NFTAI	SP500-NFTAI
0.0263	0.0074	0.0002	0.0462	−0.0204	0.0031	0.0000	−0.0635	−0.0260	0.0000	0.0348	−0.0034	−0.0001
*Band 3: 0.13 to 0.00; corresponds to infinite weeks*												
Coffee-Cotton	Coffee-Crude Oil	Coffee-Natural Gas	Coffee-Gold	Coffee-Palladium	Coffee-Platinum	Coffee-Silver	Coffee-DJI	Coffee-FTSE	Coffee-Nikkei	Coffee-SP500	Coffee-NFTAI	Cotton-Crude Oil
0.0008	0.0034	0.0059	−0.0090	0.0131	0.0000	−0.0032	0.0007	0.0002	−0.0021	0.0007	−0.0001	0.0315
Cotton-Natural Gas	Cotton-Gold	Cotton-Palladium	Cotton-Platinum	Cotton-Silver	Cotton-DJI	Cotton-FTSE	Cotton-Nikkei	Cotton-SP500	Cotton-NFTAI C	rude_Oil-Natural Gas	Crude Oil-Gold	Crude Oil-Palladium
−0.0055	−0.0063	0.0004	0.0107	0.0035	0.0325	0.0310	0.0176	0.0348	−0.0007	−0.0013	−0.0013	0.0143
Crude Oil-Platinum	Crude Oil-Silver	Crude Oil-DJI	Crude Oil-FTSE	Crude Oil-Nikkei	Crude Oil-SP500	Crude Oil-NFTAI	Natural Gas-Gold	Natural Gas-Palladium	Natural Gas-Platinum	Natural Gas-Silver	Natural Gas-DJI	Natural Gas-FTSE
0.0254	−0.0039	0.0168	0.0306	0.0318	0.0186	−0.0005	−0.0009	−0.0010	0.0002	0.0000	0.0066	−0.0010
Natural Gas-Nikkei	Natural Gas-SP500	Natural Gas-NFTAI	Gold–Palladium	Gold–Platinum	Gold–Silver	Gold-DJI	Gold-FTSE	Gold-Nikkei	Gold-SP500	Gold-NFTAI	Palladium–Platinum	Palladium–Silver
0.0094	0.0084	−0.0019	0.0067	0.0005	0.0044	−0.0002	0.0007	−0.0023	−0.0003	0.0000	0.0088	−0.0039
Palladium-DJI	Palladium-FTSE	Palladium-Nikkei	Palladium-SP500	Palladium-NFTAI	Platinum–Silver	Platinum-DJI	Platinum-FTSE	Platinum-Nikkei	Platinum-SP500	Platinum-NFTAI	Silver-DJI	Silver-FTSE
−0.0016	0.0111	0.0060	−0.0005	0.0014	−0.0057	0.0061	0.0259	0.0153	0.0074	0.0003	0.0005	0.0121
Silver-Nikkei	Silver-SP500	Silver-NFTAI	DJI-FTSE	DJI-Nikkei	DJI-SP500	DJI-NFTAI	FTSE-Nikkei	FTSE-SP500	FTSE-NFTAI	Nikkei-SP500	Nikkei-NFTAI	SP500-NFTAI
0.0073	0.0023	0.0000	0.0116	−0.0054	0.0013	0.0000	−0.0158	−0.0058	0.0000	0.0096	−0.0009	0.0000

Note: All values are in percentages. The pairwise spillover indexes show an asset's net contribution to the volatility of another asset [85].

The article "Connectedness in cross-assets and digital assets attention indices" was published in 2023. Journal: Heliyon.

**Fig. 8:** Overall rolling spillover between 12 cross-assets and NFTAI Note: Band 1 is the short-term frequency (monthly); Band 2 is the medium-term frequency (month-semi annual); Band 3 is the long-term frequency (semi-annual to infinity).

**Fig. 9:** Pairwise net rolling spillover between 12 cross-assets NFTAI Note: The pairwise spillover indexes show an asset's net contribution to the volatility of another asset [85]. The pairwise net directional connectedness is pair-specific and frequency-dependent. The pairwise net directional connectedness magnitudes vary across frequencies. Panel A is the short-term frequency (monthly); Panel B is the medium-term frequency (month-semi annual); Panel C is the long-term frequency (semi-annual to infinity).

Comparatively, when the spillover correlation (TO_ABS^a^) is picked for each index against the assets, though the spillover correlation reduce across the bands and highest at band 1, we observe from Table 4, Table 6, Table 8 that, NFTAI has the highest correlation to other assets (38.36), CBDCAI (38.36) and, ICEA has the least correlation to the assets (37.31). This is arising from the high volatility in NFT prices which has created a sense of uncertainity because investors are exposed to risk of security and credibility. Just as well, the causality spillover effect (TO_WTH^b^) follows a similar trend. This implies that though cryptocurrencies have the largest market capitalisation among digital assets, information on cryptocurrency growth does not contribute much to investors’ decisions to invest in agricultural, energy, metals and financial assets. NFTAI which is quite new in the financial markets, however, has a greater causality and correlation with assets as compared to CBDCAI and ICEA. This could be attributed to the theory of market efficiency and investor behaviour [63,65,66]. Investors may have responded to the news on cryptocurrency and heterogeneously make investment decisions based on their predictability. Though nascent, the CBDCs, it is still explorable and has not gained much attention but now NFTAI show that investors are more responsive to news on NFTs.

We find that our results are conclusively in line with [16,26,58,71,83]. We observed that the spillovers (static and rolling) are driven by short-horizons, the market is more responsive in the short-term and in the long-term, connectedness is persistent and transmitted gradually based on investor adaptiveness to the efficiency in the market. Individually, we found that crude oil was quite dominant in the spillover relation in bands 2 and 3 unlike [77] which was in the short-term and as such abrupt changes in the returns could lead to increased spillover effects [86] and are mostly receivers [32,87]. Our findings are not in line with [20] who found that the spillover of metals is high and [88] who report a large spillover from stock markets to commodities.

## 5 Conclusions

Using the frequency-domain spillover technique of [58], we explored how the connectedness between assets alters when attention indices of digital assets are integrated (CBDC, ICEA and NFT). With weekly returns of agricultural (Coffee, Cotton), energy (Crude oil, Natural gas), metals (Gold, Palladium, Platinum, Silver) and financial assets (DJI, FTSE, Nikkei, SP500), we used the wavelet technique to examine the theorised cross-asset correlation [89,75]. We found high correlations among the assets at lower and higher scales using the WMC technique and the WMCC outputs showed that DJI and SP500 dominantly in the short to semi-annual scale, had the tendency to lead or lag though in the long-run, Silver was lagging the other asset. However, because of the level of connectedness (very strong), even in the short-term, we advise investors who may be interested in diversification in these markets to be strategic [90].

The article "Connectedness in cross-assets and digital assets attention indices" was published in 2023. Journal: Heliyon.

Using Baruník-Křehlík's technique, we found that the spillover is highest at the highest frequency (Band 1) and gradually decreases across bands 2 and 3; impliclty, this is so due to impact shocks have in the short-term and how it distributes calmly in the long-run [16,58,71]. We also found that the net spillover across frequencies, for respective combinations of indices, gradually reduced and variably took turns across bands acting as net transmitter or net receiver. Dominantly, we found that Coffee, Crude oil and Gold had the most received most net spillover effects. Largely, the total spillover indices showed that NFTAI had the highest correlation and causality to other assets; followed by CBDCAI and ICEA. This was quite suprising because one would assume that with the level of market capitalisation of the cryptocurrency market and the increasing variations, ICEA would have the highest spillover index. However, based on investor behaviour to news and how efficient the market is, we observe that the NFTAI spillover indices are not far off theoretically [63,65,66]. The pairwise spillover also showed a pair-specific-frequency-dependent relationship but primarily, were highest in Bands 1 as compared to the other bands. The rolling overall and net pairwise spillovers also shows trends of reducing spillover across the bands and a pair-specific-frequency-dependent relationship respectively.

The findings of this paper would inform investors who are interested in cross-asset investments to timely and strategically create portfolios and be attentive to the market as they are higly correlated even in the short-term. Also, we recommend that with the level of high spillover across the assets and the NFTAI, investors need to be careful in the NFT market. NFTs are neither fungible nor do they have any interchangeable characteristics that would make it possible to transfer ownership and value [19,49]. Thus, with no property of mutual interchangeability, no central and authoritative body for regulating the market, investors should be wary of investing in NFTs to avoid falling victims of extreme risk from the asymmetric dynamics in the markets. Irrespective, the NFTs are distinct from other assets and could be used for diversification purposes [17,49,50,91]. Also, because of the dynamic asymmetry in the markets, investors are continually adviced to be vigilant in the markets due to incresead commodity connectedness.

The article "Connectedness in cross-assets and digital assets attention indices" was published in 2023. Journal: Heliyon.

Generally, our results have shown that there is high connectedness in cross-assets in the short-to long-term in developed and liquid markets showing how homogeneous and competitive the markets are. We have also shown that in the short-term, investors are more responsive to news in the market which reflects immediately in asset prices as compared to the medium- and long-term. This is also reflective in the Baruník-Křehlík connectedness approach where the spillover was high in the short-term. Thus, in such efficient and highly connected markets, investors should look out for hedging benefits as compared to diversification benefits. This is because of the level of risk exposure in these markets which can lead to risk. This implies that investors in the markets should be attentive to news in the when they are investing in cross-assets because there is barely any diversification benefit in the short-term. Thus, for a sustainable market, market regulators should launch policies that would maintain stabilised assets markets to prevent shocks that could come from digital assets as there is less centralisation and governance. Also, for a sustainable economic growth, the emissions from cryptocurrency and the mining of other digital assets which are built on cryptocurrencies such as NFTs, market regulators should deploy strategic measures to limit GHG emissions. Also, we found that CBCDs can provide hedging benefits to cross-assets because of its centralised and controlled effects; at different horizons, investors can recoup from ICEA but that depends on the sentiments investors as it has influence on price volatilities; and lastly, we found that NFTAI can move the price of cross-assets based on its speculative nature. Investors are however cautioned on NFTs as it is gaining more attention in the markets to note that risks in that market are still evolving and thus, it is important for thorough research before engaging in NFT investments. Also, investors are advised that based on the market dynamics, they should note that digital assets are not detached from financial assets. Thus, for effective asset allocation for a portfolio, investors must strategically analyse the market before allocating resources. Also, the findings of this study may impact policymakers’ responses to changes in various asset classes pending the level of high connectedness. Furthermore, the results of this study show heightened correlations which show significant likely interdependent risk. Thus, risk regulators should develop a framework to monitor the risk in cross-assets regularly to avoid systemic crises.

The article "Connectedness in cross-assets and digital assets attention indices" was published in 2023. Journal: Heliyon.

Theoretically, high-frequency data on asset prices provide a deeper understanding into the trends, volatility and anomalies in the dynamics of investor behaviour on the markets revealing timely decisions for investors’ decision-making process. However, this study is limited to using weekly data as opposed to high frequency data (e.g. daily data or shorter). Thus, researchers can develop daily index on digital assets attention index so that they can provide implications on high-frequency data analysis. As the case is made for increased connectedness due to financialisation of several markets, it is also becoming more and more blurry the extent of the boundaries in the different markets. For instance, given that Stable-coins are a brand of cryptocurrencies (unconventional assets) pegged to fiat currencies or relatively stable conventional assets (e.g. the US dollar) [92], the distinction between these classes of assets become fuzzy. Thus, it will be important to employ methods that can decipher these fuzzy boundaries so that investment and policy actions involving these assets are well-informed. Further, other researchers may employ computable general equilibrium (CGE) models to examine the policy actions involving these assets since they may subsequently affect expected returns and risks of assets (see, for instance, [93]). This is especially crucial since policy on these digital unconventional assets are still evolving.

## Funding

No funding was provided for this research.

## Data availability statement

The data in relation to the findings of this study are available upon request and publicly available for download at:

• https://sites.google.com/view/cryptocurrency-indices/home?authuser=0 (attention indices on Non-Fungible Tokens, Central Bank Digital Currency and cryptocurrency environmental attention)
• The financial assets (Dow Jones Industrial Average (DJI), FTSE 100 (FTSE), Nikkei 225 (Nikkei) and S&P 500 (SP500)) and commodity assets (Coffee, Cotton), energy (Crude oil, Natural Gas) and metals (Gold, Palladium, Platinum, Silver) were downloaded using the yfR package in R (https://cran.r-project.org/web/packages/yfR/index.html)

The article "Connectedness in cross-assets and digital assets attention indices" was published in 2023. Journal: Heliyon.

## CRediT authorship contribution statement

**Zynobia Barson:** Writing – review & editing, Writing – original draft, Visualization, Validation, Project administration, Investigation, Formal analysis, Conceptualization. **Peterson Owusu Junior:** Writing – review & editing, Validation, Supervision, Software, Methodology, Data curation, Conceptualization.

## Declaration of competing interest

The authors declare that they have no known competing financial interests or personal relationships that could have appeared to influence the work reported in this paper.

## List of Abbreviations

CBDC: Central Bank Digital Currency
CBDCAI: Central Bank Digital Currency Attention Index
Defi: Decentralised Finance
DJI: Dow Jones Industrial Average
FTSE: FTSE 100
GFC: Global Financial Crisis
GFEVD: Generalised Forecast Error Variance Decompositions
GHG: Greenhouse Gas
ICEA: Index On Cryptocurrency Environmental Attention
MODWT: Maximal Overlap Discrete Wavelet Transform
NFT: Non-Fungible Tokens
NFTAI: Non-Fungible Tokens Attention Index
Nikkei: Nikkei 225
SP500: S&P 500
VAR: Vector Autoregressive
WMC: Wavelet Multiple Correlation
WMCC: Wavelet Multiple Cross Correlation
